The article "A Mathematical Model Analysis for the Transmission Dynamics of Leptospirosis Disease in Human and Rodent Populations" was published in 2022. Journal: Comput Math Methods Med.

# A Mathematical Model Analysis for the Transmission Dynamics of Leptospirosis Disease in Human and Rodent Populations

**DOI:** 10.1155/2022/1806585

**Published:** 2022-09-17

**Authors:** Habtamu Ayalew Engida, David Mwangi Theuri, Duncan Gathungu, John Gachohi, Haileyesus Tessema Alemneh

**Affiliations:** ^1^Pan African University for Basic Science, Technology and Invocation (PAUSTI)/JKUAT, Kenya; ^2^Department of Mathematics, Jomo Kenyatta University of Agriculture and Technology, Kenya; ^3^Department of Public Health, Jomo Kenyatta University of Agriculture and Technology, Kenya; ^4^Department of Applied Mathematics, University of Gondar, Ethiopia

## Abstract

This work is aimed at formulating and analyzing a compartmental mathematical model to investigate the impact of rodent-born leptospirosis on the human population by considering a load of pathogenic agents of the disease in an environment and the incidence rate of human infection due to the interaction between infected rodents and the environment. Firstly, the basic properties of the model, the equilibria points, and their stability analysis are studied. We also found the basic reproduction number (*R*_0_) of the model using the next-generation matrix approach. From the stability analysis, we obtained that the disease-free equilibrium (DFE) is globally asymptotically stable if *R*_0_ < 1 and unstable otherwise. The local stability of endemic equilibrium is performed using the phenomenon of the center manifold theory, and the model exhibits forward bifurcation. The most sensitive parameters on the model outcome are also identified using the normalized forward sensitivity index. Finally, numerical simulations of the model are performed to show the stability behavior of endemic equilibrium and the varying effect of the human transmission rates, human recovery rate, and the mortality rate rodents on the model dynamics. The model is simulated using the forward fourth-order Runge-Kutta method, and the results are presented graphically. From graphical stability analysis, we observed that all trajectories of the model solutions evolve towards the unique endemic equilibrium over time when *R*_0_ > 1. Our numerical results revealed that decreasing the transmission rates and increasing the rate of recovery and reduction of the rodent population using appropriate intervention mechanisms have a significant role in reducing the spread of disease infection in the population.

## 1. Introduction

Leptospirosis is an infectious bacterial disease caused by a pathogenic spirochete bacteria called *Leptospira interrogans*, and it occurs throughout the world but is most common in tropical and subtropical regions, especially in developing countries including South-East Asia countries and sub-Sahara Africa [1–3]. It is one of the major direct zoonosis diseases worldwide that affects humans and animals [4, 5]. Recent studies reported that more than one million human cases with an estimated 60,000 deaths occur worldwide each year due to the *Leptospira interrogans* [1, 4].

The article "A Mathematical Model Analysis for the Transmission Dynamics of Leptospirosis Disease in Human and Rodent Populations" was published in 2022. Journal: Comput Math Methods Med.

Human infection occurs through direct contact with infected animal reservoir urine, tissues, or other body fluid, or more commonly by contact with infected animal (reservoirs) urine-contaminated environment [1, 6, 7]. Person-to-person transmission of the disease occurs very rarely. Globally, the main animal reservoirs of human leptospirosis are rodents (rats and mice), especially in urban slum environments [8–10]. The high concentration of Leptospira bacteria shed in slum environments mainly occurs due to the high prevalence of infection in rat population [6].

The incubation period of leptospirosis disease is typically 5 to 14 days [1, 11]. The symptoms and signs of the disease are nonfixed and may be confused with other diseases' symptoms (dengue, hantavirus, malaria, melioidosis, influenza, etc.) due to the initially nonspecific presentation. Consequently, its cases are sometimes underrecognized [11]. In humans, leptospirosis illness can be demonstrated by two stages. The primary (an acute) stage is illustrated by mild illness with nonspecific signs like higher fever, headache, and conjunctival suffusion [1, 12], while syndromes in the second (severe illness or immune) stage of leptospirosis include jaundice, kidney failure, haemorrhage (especially pulmonary), meningitis, cardiac arrhythmias, respiratory insufficiency, and hemodynamic collapse [1, 11].

Human vaccine against leptospirosis is not widely practiced and accessible only in a few developed countries which protect only against the serovar in the vaccine, and regular boosting is required [11]. However, prevention and control interventions can be implemented to avoid the risk of leptospirosis infections (especially for people whose working environment exposes them to the risk of infections), to minimize the acquisition of the infection, or to reduce the human infections in infected population. Preventive measures include personal protective equipment (PPE) (wearing rubber boots, waterproof overalls/dressings to cover wounds or skin, goggles, and rubber gloves) and personal hygiene. Environmental modifications such as draining wet areas or improvements in urban slum environment to reduce the concentration of pathogenic spirochete leptospiries from the environment [1, 12].

Patients with early leptospirosis infection (mild illness) can be treated through antibiotic doxycycline, ampicillin or amoxicillin, azithromycin, or clarithromycin. Patients with severe illness can be treated through IV penicillin and ceftriaxone drugs [1, 11].

The article "A Mathematical Model Analysis for the Transmission Dynamics of Leptospirosis Disease in Human and Rodent Populations" was published in 2022. Journal: Comput Math Methods Med.

Recently, a mathematical model has become an important tool in underlying mechanisms of disease transmission and spread and has been used to predict outcomes of diseases in communities, help to explain key factors in the disease transmission process, suggest effective control and preventive measures, and provide an estimate for the seriousness and potential scale of the epidemic [13]. In particular, deterministic mathematical models have been used to study the dynamics of infectious diseases within human and vector hosts in the population by dividing the individuals into different stages and making assumptions about the nature and time rate of transfer from one compartment to another [14].

A few researchers have been investigated a two-strain deterministic mathematical model, one strain for the human population and another strain for vectors (or animal population), for the transmission process of leptospirosis disease in various forms to demonstrate the dynamical spread of the disease between the two population groups.

Pimpunchat et al. [15] proposed the susceptible, infected, removed (SIR) model of leptospirosis which consists of both human and vector host populations. In their model, the human population is divided into three compartmental, susceptible, infected, and recovered humans, whereas the vector population was divided into two classes, susceptible and infected vectors. They performed numerical solutions to analyze and examine the behavior of the disease. Likewise, another compartmental mathematical model was developed by incorporating exposed cases in both human and vector populations for transmission dynamics of leptospirosis disease in [16]. They illustrated numerical simulations of the formulated model by using the well-known numerical method, the Runge-Kutta of fourth-order in the MATLAB program. Authors in [17] presented a compartmental mathematical model for the dynamic behavior of the leptospirosis disease with saturated incidence. They described the model using nonlinear ordinary differential equations by subdividing the host population of humans into three classes, susceptible individuals, infected individuals, and recovered individuals, and also by subdividing vectors (animal) population into two compartments, susceptible and infected vectors. They investigated the stability analysis of the disease-free and endemic equilibrium by using the basic reproduction number. From the results of stability analysis, they obtained that the disease-free equilibrium is stable both locally and globally whenever the basic reproduction number is less than one. Similarly, authors in [18] investigated a mathematical model of the leptospirosis disease using a compartmental approach. However, in view of above models, the contraction of *Leptospira interrogans* in environment for transmission had not been incorporated.

The article "A Mathematical Model Analysis for the Transmission Dynamics of Leptospirosis Disease in Human and Rodent Populations" was published in 2022. Journal: Comput Math Methods Med.

Although the human infection of the disease occurs in multiple different ways, most of the infections acquired directly or indirectly from environment (soil or water) contaminated with Leptospira especially in urban slum areas [7–9].

Motivated from [5, 17], this study examines a two-strain model, SEIRS model for the human population and another SIRS model for rodent (vector) population taking account the concentration leptospires population in environment and the transmission rates between susceptible individuals and the load of the pathogen in the environment and between susceptible rodents and infected rodents for the dynamics behavior of leptospirosis disease. Thus, in this work, we present two host populations (namely, humans and rodents) and the pathogenic population with its two growth controls (namely, the natural death rate of Leptospira and carrying capacity controls). The rest of this work is organized as follows. The leptospirosis model is described and formulated in Section 2.  Section3 is concerned with the basic properties of the model, local and global stability of disease-free equilibrium, the phenomena of bifurcation analysis, and local stability of endemic equilibrium.  Section 4 is devoted to the sensitivity analysis for the basic reproduction number (*R*_0_) of the model to each of the parameter values. The numerical simulations and discussions are presented in Section 5. Our conclusions are given in Section 6.

## 2. Model Formulation

Using system of nonlinear differential equations, we build up a compartmental mathematical model for the transmission process of leptospirosis epidemic. The model includes human, vector (rodent), and bacterial populations. The total human population denoted by *N*_*h*_(*t*) is subdivided into four compartments: *S*_*h*_(*t*), *E*_*h*_(*t*), *I*_*h*_(*t*), and *R*_*h*_(*t*). Thus,

(1) $$\begin{array}{c} N_{h}\left(t\right)=S_{h}\left(t\right)+E_{h}\left(t\right)+I_{h}\left(t\right)+R_{h}\left(t\right). \end{array}$$

The total rodent population denoted by *N*_*v*_(*t*) is subgrouped into three groups: *S*_*v*_(*t*), *I*_*v*_(*t*), and *R*_*v*_(*t*) with

(2) $$\begin{array}{c} N_{v}\left(t\right)=S_{v}\left(t\right)+I_{v}\left(t\right)+R_{v}\left(t\right). \end{array}$$

Moreover, the state variables of the model are described in Table 1.

The article "A Mathematical Model Analysis for the Transmission Dynamics of Leptospirosis Disease in Human and Rodent Populations" was published in 2022. Journal: Comput Math Methods Med.

In the formulation of the model, the following assumptions are considered:

- Each parameter of the model cannot be negative
- We assume that susceptible human and rodent populations increase at constant rates are given by recruitment of the individuals *Λ* and *Π*, respectively
- We assume that susceptible humans can be infected in two different ways: through either direct contact with infected rodents urine or contact with contaminated environments
- Assume there is a homogeneous mixing between human and rodent populations

The susceptible individuals can acquire infection with the incidence rate *λ*_*h*_ = *λ*_*hB*_ + *λ*_*hv*_ with *λ*_*hB*_ = *β*_2_*B*_*l*_/(*κ* + *B*_*l*_) and *λ*_*hv*_ = *β*_1_*I*_*v*_. The susceptible rodents can acquire infection with the force of infection *β*_3_*I*_*h*_. The population *B*_*l*_ increases its size in contaminated environment from the release of bacteria by infected humans and rodents with the rate of *τ*_1_ and *τ*_2_, respectively. Further, description of the parameters of the model is summarized in Table 2.

From the flowchart diagram in Figure 1, we obtained the following set of differential equations for the compartmental model of the leptospirosis disease.

(3) $$\begin{array}{c} \left\{\begin{array}{c} \frac{dS_{h}}{dt}=\Lambda +\gamma R_{h}-\left(\lambda_{h}+\mu \right)S_{h},\\ \frac{dE_{h}}{dt}=\lambda_{h}S_{h}-\left(\theta +\mu \right)E_{h},\\ \begin{array}{c} \frac{dI_{h}}{dt}=\theta E_{h}-\left(\alpha +\delta +\mu \right)I_{h},\\ \frac{dR_{h}}{dt}=\delta I_{h}-\left(\gamma +\mu \right)R_{h},\\ \begin{array}{c} \frac{dS_{v}}{dt}=\Pi +\rho R_{v}-\left(\beta_{3}I_{h}+\mu_{v}\right)S_{v},\\ \frac{dI_{v}}{dt}=\beta_{3}I_{h}S_{v}-\left(\sigma +\mu_{v}\right)I_{v},\\ \begin{array}{c} \frac{dR_{v}}{dt}=\sigma I_{v}-\left(\rho +\mu_{v}\right)R_{v},\\ \frac{dB_{l}}{dt}=\tau_{1}I_{h}+\tau_{2}I_{v}-\mu_{b}B_{l}, \end{array} \end{array} \end{array} \end{array}\right. \end{array}$$

where *λ*_*h*_ = *β*_2_*B*_*l*_/(*κ* + *B*_*l*_) + *β*_1_*I*_*v*_. With the initial conditions:

(4) $$\begin{array}{c} S_{h}\left(0\right)\geq 0,\\ E_{h}\left(0\right)\geq 0,\\ I_{h}\left(0\right)\geq 0,\\ R_{h}\left(0\right)\geq 0,\\ S_{v}\left(0\right)\geq 0,\\ I_{v}\left(0\right)\geq 0,\\ R_{v}\left(0\right)\geq 0,\\ B_{l}\left(0\right)\geq 0. \end{array}$$

## 3. Model Analysis

### 3.1. Positivity of Solutions

**Theorem 1 .**

Let *Ω*_*l*_(0) = (*S*_*h*_(0), *E*_*h*_(0), *I*_*h*_(0), *R*_*h*_(0), *S*_*v*_(0), *I*_*v*_(0), *R*_*v*_(0), *B*_*l*_(0)) ∈ *R*_+_^8^ ∪ {0} be the initial condition for equation (3). Then, the set of solutions {*S*_*h*_(*t*), *E*_*h*_(*t*), *I*_*h*_(*t*), *R*_*h*_(*t*), *S*_*v*_(*t*), *I*_*v*_(*t*), *R*_*v*_(*t*), *B*_*l*_(*t*)} of equation (3) is nonnegative for all *t* ≥ 0.

The article "A Mathematical Model Analysis for the Transmission Dynamics of Leptospirosis Disease in Human and Rodent Populations" was published in 2022. Journal: Comput Math Methods Med.

**Proof**

Given that a set of nonnegative initial conditions *S*_*h*_(0), *E*_*h*_(0), *I*_*h*_(0), *R*_*h*_(0), *S*_*v*_(0), *I*_*v*_(0), *R*_*v*_(0), *B*_*l*_(0), consider equation (3). Let *t*_1_ = sup{*t* > 0 : *S*_*h*_(*t*_0_) > 0, *E*_*h*_(*t*_0_) > 0, *I*_*h*_(*t*_0_) > 0, *R*_*h*_(*t*_0_) > 0, *S*_*v*_(*t*_0_) > 0, *I*_*v*_(*t*_0_) > 0, *R*_*v*_(*t*_0_) > 0, *B*_*l*_(*t*_0_) > 0, ∀*t*_0_in[0, *t*]}. From the first equation of the system (3), it follows that

(5) $$\begin{array}{c} \frac{S_{h}}{dt}+\left(\lambda_{h}\left(t\right)+\mu \right)S_{h}=\Lambda +\gamma R_{h}\left(t\right), \end{array}$$

which can be rewritten as

(6) $$\begin{array}{c} \frac{d}{dt}\left[S_{h}\left(t\right)e^{\mu t+\int_{0}^{t}\lambda_{h}\left(\tau \right)d\tau }\right]=\left(\Lambda +\gamma R_{h}\left(t\right)\right)e^{\mu t+\int_{0}^{t}\lambda_{h}\left(\tau \right)d\tau }. \end{array}$$

Thus,

(7) $$\begin{array}{c} S_{h}\left(t_{1}\right)e^{\mu t_{1}+\int_{0}^{t_{1}}\lambda_{h}\left(\tau \right)d\tau }-S_{h}\left(0\right)=\int_{0}^{t_{1}}\left(\Lambda +\gamma R_{h}\left(t\right)\right)\left[e^{\mu z+\int_{0}^{z}\lambda_{h}\left(\tau \right)d\tau }\right]dz. \end{array}$$

Therefore,

(8) $$\begin{array}{c} S_{h}\left(t_{1}\right)=S_{h}\left(0\right)e^{-\mu t_{1}-\int_{0}^{t_{1}}\lambda_{h}\left(\tau \right)d\tau }+\left[e^{-\mu t_{1}-\int_{0}^{t_{1}}\lambda_{h}\left(\tau \right)d\tau }\right]\times \int_{0}^{t_{1}}\left[e^{\mu z+\int_{0}^{z}\lambda_{h}\left(\tau \right)d\tau }\left(\Lambda +\gamma R_{h}\left(z\right)\right)\right]dz\geq 0. \end{array}$$

Similarly, the fifth equation of the system (3) yields that

(9) $$\begin{array}{c} S_{v}\left(t_{1}\right)=S_{l}\left(0\right)e^{-\mu_{l}t_{1}-\int_{0}^{t_{1}}\lambda_{l}\left(\tau \right)d\tau }+\left[e^{-\mu_{l}t_{1}-\int_{0}^{t_{1}}\lambda_{l}\left(\tau \right)d\tau }\right]\times \int_{0}^{t_{1}}\left[e^{\mu_{l}z+\int_{0}^{z}\lambda_{l}\left(\tau \right)d\tau }\left(\Pi +\rho R_{v}\left(z\right)\right)\right]dz\geq 0. \end{array}$$

Next, from the second equation of model (3), it follows that

(10) $$\begin{array}{c} \frac{dE_{h}}{dt}\geq -\left(\theta +\mu \right)E_{h}. \end{array}$$

Applying the comparison theorem and variation of formula for (10) yields

(11) $$\begin{array}{c} E_{h}\left(t\right)\geq E_{h}\left(0\right)e^{-\left(\theta +\mu \right)t}\geq 0,\forall t\geq 0. \end{array}$$

Similarly,

(12) $$\begin{array}{c} \left\{\begin{array}{c} I_{h}\left(t\right)\geq I_{h}\left(0\right)e^{-\left(\alpha +\delta +\mu \right)t}\geq 0,\forall t\geq 0,\\ R_{h}\left(t\right)\geq R_{h}\left(0\right)e^{-\left(\gamma +\mu \right)t}\geq 0,\forall t\geq 0,\\ \begin{array}{c} I_{v}\left(t\right)\geq I_{v}\left(0\right)e^{-\left(\sigma +\mu_{v}\right)t}\geq 0,\forall t\geq 0,\\ R_{v}\left(t\right)\geq R_{v}\left(0\right)e^{-\left(\rho +\mu_{v}\right)t}\geq 0,\forall t\geq 0,\\ B_{l}\left(t\right)\geq B_{l}\left(0\right)e^{-\left(\mu_{b}\right)t}\geq 0,\forall t\geq 0. \end{array} \end{array}\right. \end{array}$$

Therefore, all solutions of the system (3) remain nonnegative for all nonnegative initial conditions.

The article "A Mathematical Model Analysis for the Transmission Dynamics of Leptospirosis Disease in Human and Rodent Populations" was published in 2022. Journal: Comput Math Methods Med.

### 3.2. Invariant Region

**Theorem 2 .**

All solutions of the leptospirosis model equation (3) remain in *Ω*_*l*_ = {(*S*_*h*_, *E*_*h*_, *I*_*h*_, *R*_*h*_, *S*_*v*_, *I*_*v*_, *R*_*v*_, *B*_*l*_) ∈ *R*_+_^8^ : 0 ≤ *N*_*h*_(*t*) ≤ *Λ*/*μ*, 0 ≤ *N*_*v*_(*t*) ≤ *Π*/*μ*_*v*_, 0 ≤ *B*_*l*_(*t*) ≤ *τ*^∗^/*μ*_*bl*_((*Λ*/*μ*) + (*Π*/*μ*_*v*_))}.

**Proof**

From equation (1), we get

(13) $$\begin{array}{c} \frac{dN_{h}}{dt}=\frac{dS_{h}}{dt}+\frac{dE_{h}}{dt}+\frac{dI_{h}}{dt}+\frac{dR_{h}}{dt}. \end{array}$$

The first four equations of the system (3) and equation (13) give rise to

(14) $$\begin{array}{c} \frac{dN_{h}}{dt}=\Lambda -\mu N_{h}-\alpha I_{h}. \end{array}$$

Since the parameter, *α*, and the state variable *I*_*h*_ are nonnegative in (14), we have

(15) $$\begin{array}{c} \frac{dN_{h}}{dt}\leq \Lambda -\mu N_{h}. \end{array}$$

Let *N*_*h*_^∗^(*t*) be the solution of the ODE *dN*_*h*_/*dt* = *Λ* − *μN*_*h*_ with an initial condition. Then,

(16) $$\begin{array}{c} \frac{dN_{h}^{*}}{dt}=\Lambda -\mu N_{h}^{*}\text{ with }N_{h}^{*}\left(0\right)=N_{h0}^{*}\forall t\geq 0. \end{array}$$

Thus, equation (16) has a unique solution. By applying separation of variable on the differential equation (16), we get

(17) $$\begin{array}{c} \frac{dN_{h}^{*}}{\Lambda -\mu N_{h}^{*}}=dt. \end{array}$$

Integrating (17) on both sides yields

(18) $$\begin{array}{c} N_{h}^{*}\left(t\right)=N_{h}^{*}\left(0\right)e^{-\mu t}+\frac{\Lambda }{\mu }\left(1-e^{-\mu t}\right). \end{array}$$

We now apply the comparison theorem [19] on the differential equation (15) and then *N*_*h*_(*t*) ≤ *N*_*h*_^∗^(*t*). Thus,

(19) $$\begin{array}{c} N_{h}\left(t\right)\leq N_{h}^{*}\left(0\right)e^{-\mu t}+\frac{\Lambda }{\mu }\left(1-e^{-\mu t}\right). \end{array}$$

As *t*⟶∞, the population size *N*_*h*_⟶*Λ*/*μ*.

Hence,

(20) $$\begin{array}{c} N_{h}\left(t\right)\leq \frac{\Lambda }{\mu }\text{ for }0\leq N_{h}^{*}\left(0\right)\leq \frac{\Lambda }{\mu },\forall t\geq 0. \end{array}$$

On the other hand, if *N*_*h*_^∗^(0) > *Λ*/*μ*, the solution decrease to *Λ*/*μ* as *t*⟶∞.

Also, the last equation of (3) and equations (20) and (23) imply that

(21) $$\begin{array}{c} \frac{dB_{l}}{dt}\leq \tau^{*}\left(\frac{\Lambda }{\mu }+\frac{\Pi }{\mu_{v}}\right)-\mu_{b}B_{l}, \end{array}$$

where *τ*^∗^ = max{*τ*_1_, *τ*_2_}.

The article "A Mathematical Model Analysis for the Transmission Dynamics of Leptospirosis Disease in Human and Rodent Populations" was published in 2022. Journal: Comput Math Methods Med.

Equation (21) yields

(22) $$\begin{array}{c} B_{l}\left(t\right)\leq B_{l}\left(0\right)e^{-\mu_{bl}t}+\frac{\tau^{*}}{\mu_{bl}}\left(\frac{\Lambda }{\mu }+\frac{\Pi }{\mu_{v}}\right)\left(\left(1-e^{-\mu_{b}t}\right)\right)\forall t\geq 0. \end{array}$$

Hence,

(23) $$\begin{array}{c} \Omega_{h}=\left\{\left(S_{h},E_{h},I_{h},R_{h},B_{l}\right)\in R_{+}^{5}:0\leq N_{h}\left(t\right)\leq \frac{\Lambda }{\mu },0\leq B_{l}\leq \frac{\tau^{*}}{\mu_{bl}}\left(\frac{\Lambda }{\mu }+\frac{\Pi }{\mu_{v}}\right)\right\}, \end{array}$$

is positively invariant region.

Finally, the 5th equation of (3) implies that

(24) $$\begin{array}{c} \frac{dN_{v}}{dt}\leq \Pi -\mu N_{v},\text{with }N_{v}\left(0\right)=N_{v,0}. \end{array}$$

Then, equation (24) has a unique solution. Similarly, applying the comparison theorem and integrating the differential equation (21) yield

(25) $$\begin{array}{c} N_{v}\left(t\right)=N_{v}\left(0\right)e^{-\mu_{v}t}+\frac{\pi }{\mu_{v}}\left(1-e^{-\mu_{v}t}\right). \end{array}$$

Therefore,

(26) $$\begin{array}{c} 0\leq N_{v}\left(t\right)\leq \frac{\Pi }{\mu_{v}}\text{ for }0\leq N_{v}\left(0\right)\leq \frac{\Pi }{\mu_{v}},\\ \Omega_{v}=\left\{\left(S_{v},I_{v},R_{v}\right)\in R_{+}^{3}:0\leq N_{v}\left(t\right)\leq \frac{\Pi }{\mu_{v}}\right\}. \end{array}$$

Therefore, the biologically feasible region for (3) is given by

(27) $$\begin{array}{c} \Omega_{l}=\Omega_{h}\times \Omega_{v}\subset R_{+}^{5}\times R_{+}^{3}. \end{array}$$

Therefore, every solution of the differential equation model with initial conditions in *Ω*_*l*_ remains in *Ω*_*l*_∀*t* ≥ 0. Thus, the region *Ω*_*l*_ is positively invariant with respect to the system (3).

### 3.3. Disease-Free Equilibrium

The disease-free equilibrium (DFE) of the model (3) only exists in the absence of infections. We compute DFE by setting left-hand side of the system (3) equal to zero. Since *E*_*h*_^∗^ = *I*_*h*_^∗^ = *R*_*h*_^∗^ = *I*_*v*_^∗^ = *R*_*v*_^∗^ = *B*_*l*_^∗^ = 0 at DFE, we have

(28) $$\begin{array}{c} \left\{\begin{array}{c} \Lambda +\gamma R_{h}^{*}-\left(\frac{\beta_{1}B_{l}^{*}}{\kappa +B_{l}^{*}}+\beta_{2}I_{v}^{*}+\mu \right)S_{h}^{*}=0,\\ \Pi +\rho R_{v}^{*}-\left(\beta_{3}I_{l}^{*}+\mu_{v}\right)S_{v}^{*}=0. \end{array}\right. \end{array}$$

Thus, the system (28) yields *S*_*h*_^∗^ = *Λ*/*μ* and *S*_*v*_^∗^ = *Π*/*μ*_*v*_. Therefore, the DFE point of the model (3) is given by

(29) $$\begin{array}{c} \varepsilon_{0l}^{*}=\left(S_{h}^{*},0,0,0,S_{v}^{*},0,0,0\right)=\left(\frac{\Lambda }{\mu },0,0,0,\frac{\Pi }{\mu_{v}},0,0,0\right). \end{array}$$

To compute the basic reproduction number for our model (3), we follow the method presented in [20]. Considering only the infective compartments *W* = (*E*_*h*_, *I*_*h*_, *I*_*v*_, *B*_*l*_) in (3), then we have *dW*/*dt* = *F*(*t*) − *V*(*t*),

(30) $$\begin{array}{c} F\left(t\right)=\left[\begin{array}{c} \lambda_{h}S_{h}\\ 0\\ \beta_{3}S_{v}I_{h}\\ 0 \end{array}\right],\\ V\left(t\right)=\left[\begin{array}{c} \varepsilon_{1}E_{h}\\ -\theta E_{h}+\varepsilon_{2}I_{h}\\ \varepsilon_{4}I_{v}\\ -\tau_{1}I_{h}-\tau_{2}I_{v}+\mu_{bl}B_{l} \end{array}\right], \end{array}$$

where

(31) $$\begin{array}{c} \lambda_{h}=\frac{\beta_{2}B_{l}}{\kappa +B_{l}}+\beta_{1}I_{v},\\ \varepsilon_{1}=\theta +\mu ,\\ \varepsilon_{2}=\alpha +\delta +\mu , \end{array}$$

The Jacobian matrices of *F*(*t*) and of *V*(*t*) at *ε*_0*l*_^∗^ are, respectively, given by

(32) $$\begin{array}{c} F=\left[\begin{array}{cccc} 0 & 0 & \frac{\beta_{1}\Lambda }{\mu } & \frac{\beta_{2}\Pi }{\mu \kappa }\\ 0 & 0 & 0 & 0\\ 0 & \frac{\beta_{3}\Pi }{\mu_{v}} & 0 & 0\\ 0 & 0 & 0 & 0 \end{array}\right],\\ V=\left[\begin{array}{cccc} \varepsilon_{1} & 0 & 0 & 0\\ -\theta & \varepsilon_{2} & 0 & 0\\ 0 & 0 & \varepsilon_{3} & 0\\ 0 & -\tau_{1} & -\tau_{2} & \mu_{b} \end{array}\right]. \end{array}$$

Therefore, the next-generation matrix of the model is given by

(33) $$\begin{array}{c} 3G=FV^{-1}=\left[\begin{array}{cccc} 0 & 0 & \frac{\beta_{1}\Lambda }{\mu } & \frac{\beta_{2}\Lambda }{\mu \kappa }\\ 0 & 0 & 0 & 0\\ 0 & \frac{\beta_{3}\Pi }{\mu_{v}} & 0 & 0\\ 0 & 0 & 0 & 0 \end{array}\right]\left[\begin{array}{cccc} \frac{1}{\varepsilon_{1}} & 0 & 0 & 0\\ \frac{\theta }{\varepsilon_{1}\varepsilon_{2}} & \frac{1}{\varepsilon_{2}} & 0 & 0\\ 0 & 0 & \frac{1}{\varepsilon_{4}} & 0\\ \frac{\theta \tau_{1}}{\varepsilon_{1}\varepsilon_{2}\mu_{b}} & \frac{\tau_{1}}{\varepsilon_{2}\mu_{b}} & \frac{\tau_{2}}{\varepsilon_{4}\mu_{b}} & \frac{1}{\mu_{b}} \end{array}\right]=\left[\begin{array}{cccc} y_{1} & y_{2} & y_{3} & y_{4}\\ 0 & 0 & 0 & 0\\ y_{5} & y_{6} & 0 & 0\\ 0 & 0 & 0 & 0 \end{array}\right], \end{array}$$

where

(34) $$\begin{array}{c} y_{1}=\frac{\beta_{2}\Lambda \theta \tau_{1}}{\kappa \mu \mu_{b}\varepsilon_{1}\varepsilon_{2}},\\ y_{2}=\frac{\beta_{2}\Lambda \tau_{1}}{\kappa \mu \mu_{b}\varepsilon_{2}},\\ y_{3}=\frac{\Lambda \left(\beta_{2}\tau_{2}+\beta_{1}\kappa \mu_{b}\right)}{\kappa \mu \mu_{b}\varepsilon_{4}},\\ y_{4}=\frac{\beta_{2}\Lambda }{\kappa \mu \mu_{b}},\\ y_{5}=\frac{\beta_{3}\Pi \theta }{\mu_{v}\varepsilon_{1}\varepsilon_{2}},\\ y_{6}=\frac{\beta_{3}\Pi }{\mu_{v}\varepsilon_{2}}. \end{array}$$

Considering |*G* − *λI*| = 0, we have

(35) $$\begin{array}{c} \left|\begin{array}{cccc} y_{1}-\lambda & y_{2} & y_{3} & y_{4}\\ 0 & -\lambda & 0 & 0\\ y_{5} & y_{6} & -\lambda & 0\\ 0 & 0 & 0 & -\lambda \end{array}\right|=0⟹\lambda^{2}\left(\lambda^{2}-\lambda y_{1}-y_{3}y_{5}\right)=0. \end{array}$$

Thus,

(36) $$\begin{array}{c} \lambda_{1}=\lambda_{2}=0,\\ \lambda_{3}=\frac{1}{2}\left(y_{1}-\sqrt{y_{1}^{2}+4y_{3}y_{5}}\right)<0,\\ \lambda_{4}=\frac{1}{2}\left(y_{1}+\sqrt{y_{1}^{2}+4y_{3}y_{5}}\right)>0, \end{array}$$

are the eigenvalues of the matrix *G*. Therefore, the basic reproduction number of the model is given by

(37) $$\begin{array}{c} R_{0}=\rho \left(G\right)=\frac{1}{2}\left(\frac{\beta_{2}\Lambda \theta \tau_{1}}{\kappa \mu \mu_{b}\varepsilon_{1}\varepsilon_{2}}+\sqrt{{\left(\frac{\beta_{2}\Lambda \theta \tau_{1}}{\kappa \mu \mu_{b}\varepsilon_{1}\varepsilon_{2}}\right)}^{2}+4\frac{\beta_{3}\Pi \Lambda \theta \left(\beta_{2}\tau_{2}+\beta_{1}\kappa \mu_{b}\right)}{\kappa \mu \mu_{v}\mu_{b}\varepsilon_{1}\varepsilon_{2}\varepsilon_{4}}}\right). \end{array}$$

The basic reproduction number *R*_0_ can be written in terms of the basic reproduction numbers corresponding to the vector transmission *R*_*v*_, human transmission *R*_*h*_, and environment-to-human transmission *R*_*b*_ as

(38) $$\begin{array}{c} R_{0}=\frac{1}{2}\left[R_{b}+\sqrt{R_{b}^{2}+4R_{hv}}\right], \end{array}$$

where *R*_*b*_ = *β*_2_*Λθτ*_1_/*κμμ*_*b*_*ε*_1_*ε*_2_ and *R*_*hv*_ = *R*_*h*_ + *R*_*v*_ with *R*_*h*_ = *β*_3_*β*_2_*ΠΛθτ*_2_/*κμμ*_*v*_*μ*_*b*_*ε*_1_*ε*_2_*ε*_4_ and *R*_*v*_ = *β*_3_*β*_1_*ΠΛθ*/*μμ*_*v*_*ε*_1_*ε*_2_*ε*_4_.

The article "A Mathematical Model Analysis for the Transmission Dynamics of Leptospirosis Disease in Human and Rodent Populations" was published in 2022. Journal: Comput Math Methods Med.

### 3.4. Local Stability of the Disease-Free Equilibrium

**Theorem 3 .**

The disease-free equilibrium point, *ε*_0*l*_^∗^, is locally asymptotically stable whenever *R*_0_ < 1 and unstable otherwise.

**Proof**

The Jacobian matrices of the model (3) at DFE *ε*_0*l*_^∗^ is given by

(39) $$\begin{array}{c} J\left(\varepsilon_{0l}^{*}\right)=\left[\begin{array}{cccccccc} -\mu & 0 & 0 & \gamma & 0 & \frac{-\beta_{1}\Lambda }{\mu } & 0 & \frac{-\beta_{2}\Lambda }{\mu \kappa }\\ 0 & -\varepsilon_{1} & 0 & 0 & 0 & \frac{\beta_{1}\Lambda }{\mu } & 0 & \frac{\beta_{2}\Lambda }{\mu \kappa }\\ 0 & \theta & -\varepsilon_{2} & 0 & 0 & 0 & 0 & 0\\ 0 & 0 & \delta & -\varepsilon_{3} & 0 & 0 & 0 & 0\\ 0 & 0 & \frac{-\beta_{3}\Pi }{\mu_{v}} & 0 & -\mu_{v} & 0 & \rho & 0\\ 0 & 0 & \frac{\beta_{3}\Pi }{\mu_{v}} & 0 & 0 & -\varepsilon_{4} & 0 & 0\\ 0 & 0 & 0 & 0 & 0 & \sigma & -\varepsilon_{5} & 0\\ 0 & 0 & \tau_{1} & 0 & 0 & \tau_{2} & 0 & -\mu_{b} \end{array}\right], \end{array}$$

where *ε*_1_ = *θ* + *μ*, *ε*_2_ = *α* + *δ* + *μ*, *ε*_3_ = *γ* + *μ*, *ε*_4_ = *σ* + *μ*_*v*_, and *ε*_5_ = *ρ* + *μ*_*v*_.

Expanding the determinant of the characteristic equation |*J*(*ε*_0*l*_^∗^) − *λI*| = 0 by the first, fourth, fifth, and seventh columns, respectively, we obtain four of the eigenvalues of *J*(*ε*_0*l*_^∗^): *λ*_1_ = −*μ*, *λ*_2_ = −(*γ* + *μ*), *λ*_3_ = −*μ*_*v*_and*λ*_4_ = −(*ρ* + *μ*_*v*_). The other four eigenvalues will be determined from the following polynomial equation:

(40) $$\begin{array}{c} \left|\begin{array}{cccc} -\varepsilon_{1}-\lambda & 0 & \frac{\beta_{1}\Lambda }{\mu } & \frac{\beta_{2}\Lambda }{\mu \kappa }\\ \theta & -\varepsilon_{2}-\lambda & 0 & 0\\ 0 & \frac{\beta_{3}\Pi }{\mu_{v}} & -\varepsilon_{4}-\lambda & 0\\ 0 & \tau_{1} & \tau_{2} & -\mu_{b}-\lambda \end{array}\right|=0,\\ ⟹P_{4}\left(\lambda \right)=\lambda^{4}+A_{1}\lambda^{3}+A_{2}\lambda^{2}+A_{3}\lambda +A_{4}=0, \end{array}$$

where

(41) $$\begin{array}{c} A_{1}=\varepsilon_{1}+\varepsilon_{2}+\varepsilon_{4}+\mu_{b},\\ A_{2}=\varepsilon_{1}\mu_{b}+\varepsilon_{1}\varepsilon_{2}+\varepsilon_{1}\varepsilon_{4}+\varepsilon_{2}\mu_{b}+\varepsilon_{4}\mu_{b}+\varepsilon_{2}\varepsilon_{4},\\ A_{3}=\varepsilon_{1}\varepsilon_{2}\mu_{b}+\varepsilon_{1}\varepsilon_{4}\mu_{b}+\varepsilon_{1}\varepsilon_{2}\varepsilon_{4}+\varepsilon_{2}\varepsilon_{4}\mu_{b}-\frac{\beta_{2}\Lambda \tau_{1}\theta }{\mu \kappa }-\frac{\beta_{1}\beta_{3}\Lambda \Pi \theta }{\mu \mu_{v}}=\varepsilon_{4}\mu_{b}\left(\varepsilon_{1}+\varepsilon_{2}\right)+\varepsilon_{1}\varepsilon_{2}\mu_{b}\left(1-\frac{\beta_{2}\Lambda \theta \tau_{1}}{\kappa \mu \mu_{b}\varepsilon_{1}\varepsilon_{2}}\right)+\varepsilon_{1}\varepsilon_{2}\varepsilon_{4}\left(1-\frac{\beta_{1}\beta_{3}\Lambda \Pi \theta }{\mu \mu_{v}\varepsilon_{1}\varepsilon_{2}\varepsilon_{4}}\right)=\varepsilon_{4}\mu_{b}\left(\varepsilon_{1}+\varepsilon_{2}\right)+\varepsilon_{1}\varepsilon_{2}\mu_{b}\left(1-R_{b}\right)+\varepsilon_{1}\varepsilon_{2}\varepsilon_{4}\left(1-R_{v}\right),\\ A_{4}=\varepsilon_{1}\varepsilon_{2}\varepsilon_{4}\mu_{b}-\left(\frac{\beta_{2}\Lambda \theta \tau_{1}\varepsilon_{4}}{\mu \kappa }+\frac{\beta_{1}\beta_{3}\Lambda \Pi \theta \mu_{b}}{\mu \mu_{v}}+\frac{\beta_{2}\beta_{3}\Lambda \Pi \theta \tau_{2}}{\kappa \mu \mu_{v}}\right)=\varepsilon_{1}\varepsilon_{2}\varepsilon_{4}\mu_{b}-\left(\frac{\beta_{2}\Lambda \theta \tau_{1}\varepsilon_{4}}{\mu \kappa }+\frac{\beta_{3}\Pi \Lambda \theta \left(\beta_{2}\tau_{2}+\beta_{1}\kappa \mu_{b}\right)}{\kappa \mu \mu_{v}}\right)=\varepsilon_{1}\varepsilon_{2}\varepsilon_{4}\mu_{b}\left[1-\left(\frac{\beta_{2}\Lambda \theta \tau_{1}\varepsilon_{4}}{\mu \kappa }+\frac{\beta_{3}\Pi \Lambda \theta \left(\beta_{2}\tau_{2}+\beta_{1}\kappa \mu_{b}\right)}{\kappa \mu \mu_{v}}\right)\right]=\varepsilon_{1}\varepsilon_{2}\varepsilon_{4}\mu_{b}\left[1-\left(R_{b}+R_{hv}\right)\right]. \end{array}$$

Since all the model parameters are positive, the above four eigenvalues of the matrix *J*(*ε*_0*l*_^∗^) are negative real numbers. To ensure that all the remaining four eigenvalues of the matrix have negative real parts, the Routh-Hurwitz stability criterion (see Theorem 5.1 in [21]) requires *A*_1_ > 0, *A*_2_ > 0, *A*_3_ > 0, *A*_4_ > 0, *A*_1_*A*_2_ − *A*_3_ > 0, and *A*_1_*A*_2_*A*_3_ − (*A*_3_^2^ + *A*_1_^2^*A*_4_) > 0. Among these, *A*_1_ > 0 and *A*_2_ > 0 are obvious.

The article "A Mathematical Model Analysis for the Transmission Dynamics of Leptospirosis Disease in Human and Rodent Populations" was published in 2022. Journal: Comput Math Methods Med.

Similarly,

(42) $$\begin{array}{c} A_{1}A_{2}-A_{3}=A_{2}\left(\varepsilon_{4}+\mu_{b}\right)+\varepsilon_{2}^{2}\left(\varepsilon_{1}+\varepsilon_{4}+\mu_{b}\right)+\varepsilon_{1}\left(\varepsilon_{1}\mu_{b}+\varepsilon_{1}\varepsilon_{2}+\varepsilon_{2}\mu_{b}+\varepsilon_{1}\varepsilon_{4}+\varepsilon_{2}\varepsilon_{4}\right)+\frac{\beta_{2}\Lambda \tau_{1}\theta }{\mu \kappa }+\frac{\beta_{1}\beta_{3}\Lambda \Pi \theta }{\mu \mu_{v}}>0. \end{array}$$

The other three inequalities hold when *R*_0_ > 1; the details are described as follows.

Since *R*_*b*_ < *R*_0_, 1 − *R*_*b*_ > 0 for *R*_0_ < 1. Similarly, 1 − *R*_*v*_ = (1 − *R*_0_)[1 − *R*_*b*_ + *R*_0_] + *R*_*b*_ + *R*_*h*_ > 0 for *R*_0_ < 1. Thus,

(43) $$\begin{array}{c} A_{3}=\varepsilon_{4}\mu_{b}\left(\varepsilon_{1}+\varepsilon_{2}\right)+\varepsilon_{1}\varepsilon_{2}\mu_{b}\left(1-R_{b}\right)+\varepsilon_{1}\varepsilon_{2}\varepsilon_{4}\left(1-R_{v}\right)>0\text{ if }R_{0}<1. \end{array}$$

Next,

(44) $$\begin{array}{c} A_{4}=\varepsilon_{1}\varepsilon_{2}\varepsilon_{4}\mu_{b}\left[1-\left(R_{b}+R_{hv}\right)\right]=\varepsilon_{1}\varepsilon_{2}\varepsilon_{4}\mu_{b}\left(1-R_{0}\right)\left[1-R_{b}+R_{0}\right]>0\text{ if }R_{0}<1. \end{array}$$

Finally, we need to show that *A*_1_*A*_2_*A*_3_ − (*A*_3_^2^ + *A*_1_^2^*A*_4_) > 0. Let

(45) $$\begin{array}{c} \phi_{0}=\varepsilon_{1}\mu_{b},\\ \phi_{1}=\varepsilon_{1}\varepsilon_{2},\\ \phi_{2}=\varepsilon_{1}\varepsilon_{4},\\ \phi_{3}=\varepsilon_{2}\mu_{b},\\ \phi_{4}=\varepsilon_{4}\mu_{b},\\ \phi_{5}=\varepsilon_{2}\varepsilon_{4},\\ \psi_{0}=\varepsilon_{4}\mu_{b}\left(\varepsilon_{1}+\varepsilon_{2}\right),\\ \psi_{1}=\varepsilon_{1}\varepsilon_{2}\mu_{b}\left(1-R_{b}\right),\\ \psi_{3}=\varepsilon_{1}\varepsilon_{2}\varepsilon_{4}\left(1-R_{v}\right). \end{array}$$

Then, *A*_2_ = *ϕ*_0_ + *ϕ*_1_ + *ϕ*_2_ + *ϕ*_3_ + *ϕ*_4_ + *ϕ*_5_, and *A*_3_ = *ψ*_0_ + *ψ*_1_ + *ψ*_2_.

Now,

(46) $$\begin{array}{c} A_{1}A_{2}A_{3}=\varepsilon_{1}\left[\psi_{0}\left(\phi_{0}+\phi_{1}+\phi_{2}+\phi_{3}+\phi_{4}+\phi_{5}\right)+\psi_{1}\left(\phi_{0}+\phi_{1}+\phi_{2}+\phi_{3}+\phi_{4}+\phi_{5}\right)+\psi_{2}\left(\phi_{0}+\phi_{1}+\phi_{2}+\phi_{3}+\phi_{4}+\phi_{5}\right)\right]+\varepsilon_{2}\left[\psi_{0}\left(\phi_{0}+\phi_{1}+\phi_{2}+\phi_{3}+\phi_{4}+\phi_{5}\right)+\psi_{1}\left(\phi_{0}+\phi_{1}+\phi_{2}+\phi_{3}+\phi_{4}+\phi_{5}\right)+\psi_{2}\left(\phi_{0}+\phi_{1}+\phi_{2}+\phi_{3}+\phi_{4}+\phi_{5}\right)\right]+\varepsilon_{4}\left[\psi_{0}\left(\phi_{0}+\phi_{1}+\phi_{2}+\phi_{3}+\phi_{4}+\phi_{5}\right)+\psi_{1}\left(\phi_{0}+\phi_{1}+\phi_{2}+\phi_{3}+\phi_{4}+\phi_{5}\right)+\psi_{2}\left(\phi_{0}+\phi_{1}+\phi_{2}+\phi_{3}+\phi_{4}+\phi_{5}\right)\right]+\mu_{b}\left[\psi_{0}\left(\phi_{0}+\phi_{1}+\phi_{2}+\phi_{3}+\phi_{4}+\phi_{5}\right)+\psi_{1}\left(\phi_{0}+\phi_{1}+\phi_{2}+\phi_{3}+\phi_{4}+\phi_{5}\right)+\psi_{2}\left(\phi_{0}+\phi_{1}+\phi_{2}+\phi_{3}+\phi_{4}+\phi_{5}\right)\right],\\ A_{3}^{2}+A_{1}^{2}A_{4}={\left(\psi_{0}+\psi_{1}+\psi_{2}\right)}^{2}+{\left(\varepsilon_{1}+\varepsilon_{2}+\varepsilon_{4}+\mu_{b}\right)}^{2}\varepsilon_{1}\varepsilon_{2}\varepsilon_{4}\mu_{b}\left[1-R_{b}-R_{hv}\right]=\psi_{0}^{2}+\psi_{1}^{2}+\psi_{2}^{2}+2\left(\psi_{0}\psi_{1}+\psi_{0}\psi_{2}+\psi_{1}\psi_{2}\right)+\left[\varepsilon_{1}^{2}+\varepsilon_{2}^{2}+\varepsilon_{4}^{2}+\mu_{b}^{2}+2\left(\varepsilon_{1}\varepsilon_{2}+\varepsilon_{1}\varepsilon_{4}+\varepsilon_{1}\mu_{b}+\varepsilon_{2}\varepsilon_{4}+\varepsilon_{2}\mu_{b}+\varepsilon_{4}\mu_{b}\right)\right]\varepsilon_{1}\varepsilon_{2}\varepsilon_{4}\mu_{b}\left[1-R_{b}-R_{hv}\right]. \end{array}$$

After manipulating the parameters algebraically, we obtain

(47) $$\begin{array}{c} A_{1}A_{2}A_{3}-\left(A_{3}^{2}+A_{1}^{2}A_{4}\right)=\Omega_{0}+\Omega_{1}, \end{array}$$

where

(48) $$\begin{array}{c} \Omega_{0}=\varepsilon_{1}\left[\psi_{0}\left(\phi_{0}+\phi_{1}+\phi_{2}+\phi_{4}\right)+\psi_{1}\left(\phi_{0}+\phi_{1}+\phi_{4}\right)+\psi_{2}\left(\phi_{1}+\phi_{2}+\phi_{4}\right)\right]+\varepsilon_{2}\left[\psi_{1}\left(\phi_{0}+\phi_{1}+\phi_{2}+\phi_{3}+\phi_{4}\right)+\psi_{2}\left(\phi_{0}+\phi_{1}+\phi_{2}+\phi_{4}+\phi_{5}\right)\right]+\varepsilon_{4}\left[\psi_{0}\left(\phi_{1}+\phi_{2}+\phi_{4}\right)+\psi_{2}\left(\phi_{1}+\phi_{2}+\phi_{4}+\phi_{5}\right)\right]+\mu_{b}\left[\psi_{0}\left(\phi_{2}+\phi_{3}+\phi_{4}+\phi_{5}\right)+\psi_{1}\left(\phi_{0}+\phi_{1}+\phi_{2}+\phi_{3}+\phi_{4}+\phi_{5}\right)>0\right],\\ \Omega_{1}=\varepsilon_{1}\left[\phi_{3}R_{b}\left(A_{3}+\psi_{0}\right)+\phi_{5}A_{3}R_{v}\right]+\left[\left(\varepsilon_{1}^{2}+\varepsilon_{2}^{2}+A_{2}\right)\right.\phi_{1}\phi_{4}\left(1+R_{h}\right)+\phi_{4}\left(\phi_{5}^{2}+\phi_{0}^{2}+\varepsilon_{2}A_{2}\right)+\left(\varepsilon_{4}^{2}+\mu_{b}^{2}+A_{2}\right)\phi_{1}\phi_{4}\left(R_{b}+R_{hv}\right)>0. \end{array}$$

Clearly, *Ω*_0_ > 0 and *Ω*_1_ > 0.

The article "A Mathematical Model Analysis for the Transmission Dynamics of Leptospirosis Disease in Human and Rodent Populations" was published in 2022. Journal: Comput Math Methods Med.

Therefore, *A*_1_*A*_2_*A*_3_ − (*A*_3_^2^ + *A*_1_^2^*A*_4_) > 0 if *R*_0_ < 1. This completes the proof.

### 3.5. Global Stability of the Disease-Free Equilibrium

The method illustrated in [22, 23] is used to investigate the global asymptotic stability (GAS) of DFE point of the model. Firstly, the model (3) must be written in the form:

(49) $$\begin{array}{c} \left\{\begin{array}{c} \frac{dX}{dt}=F\left(X,Y\right),\\ \frac{dY}{dt}=G\left(X,Y\right),G\left(X,0\right)=0. \end{array}\right. \end{array}$$

where *X* = (*S*_*h*_, *R*_*h*_, *S*_*v*_, *R*_*v*_) represents the number of uninfected individuals and *Y* = (*E*_*h*_, *I*_*h*_, *I*_*v*_, *B*_*l*_) denotes the number of infected individuals. Let *X*^∗^ be the disease-free equilibrium of the system *dX*/*dt* = *F*(*X*, 0). Then, *X*^∗^ = (*Λ*/*μ*, 0, *Π*/*μ*_*v*_, 0). The DFE point of the model *ε*_0*l*_^∗^ = (*X*^∗^, 0) = (*Λ*/*μ*, 0, 0, 0, *Π*/*μ*_*v*_, 0, 0, 0) is guaranteed to be GAS if *R*_0_ < 1 (which is locally asymptotically stable (LAS)), and the following two conditions H_1_ and H_2_ hold:

H_1_: For *dX*/*dt* = *F*(*X*, 0), *X*^∗^ is globally asymptotically stable.

H_2_: *G*(*X*, *Y*) = *AY* − *G*^⋆^(*X*, *Y*), *G*^⋆^(*X*, *Y*) ≥ 0, ∀(*X*, *Y*) ∈ *Ω*_*l*_, where *A* = *∂G*(*ε*_0*l*_^∗^)/*∂Y* is an *M*-matrix and *Ω*_*l*_ is the region where the model makes biological sense. If the model equation (3) satisfies the above two conditions, then the following theorem holds.

**Theorem 4 .**

The disease-free equilibrium point, *ε*_0*l*_^∗^ = (*Λ*/*μ*, 0, 0, 0, *Π*/*μ*_*v*_, 0, 0, 0), is GAS for the model (3) provided that *R*_0_ < 1 (LAS) and conditions H_1_ and H_2_ hold.

**Proof**

We only need to show that the conditions H_1_ and H_2_ hold when *R*_0_ < 1. Considering the system (3), we have

(50) $$\begin{array}{c} F\left(X,0\right)=\left[\begin{array}{c} S_{h\prime }\left(t\right)\\ R_{h\prime }\left(t\right)\\ S_{v\prime }\left(t\right)\\ R_{v\prime }\left(t\right) \end{array}\right]=\left[\begin{array}{c} \Lambda +\gamma R_{h}-\mu S_{h}\\ -\left(\gamma +\mu \right)R_{h}\\ \Pi +\rho R_{v}-\mu_{v}S_{v}\\ -\left(\rho +\mu_{v}\right)R_{v} \end{array}\right],X^{*}=\left(\frac{\Lambda }{\mu },0,\frac{\Pi }{\mu_{v}},0\right). \end{array}$$

Note that the second and the fourth equations of the system (50) are first-order linear ODEs, and their solutions are given by, respectively,

(51) $$\begin{array}{c} R_{h}\left(t\right)=R_{h,0}e^{-\left(\gamma +\mu \right)t}, \end{array}$$

(52) $$\begin{array}{c} R_{v}\left(t\right)=R_{v,0}e^{-\left(\rho +\mu_{v}\right)t}. \end{array}$$

Comparing equation (51) and the first equation of the system (50) yields

(53) $$\begin{array}{c} S\prime_{h}\left(t\right)=\Lambda +\gamma R_{v,0}e^{-\left(\rho +\mu_{v}\right)}-\mu S_{h}\left(t\right). \end{array}$$

Solving the first-order linear ODE (53), its solution is found as

(54) $$\begin{array}{c} S_{h}\left(t\right)=\frac{\Lambda }{\mu }+S_{h,0}e^{-\mu t}-R_{h,0}e^{-\left(\gamma +\mu \right)t}. \end{array}$$

Similarly,

(55) $$\begin{array}{c} S_{v}^{\prime }\left(t\right)=\Pi +\rho R_{v,0}e^{-\left(\rho +\mu_{v}\right)t}-\mu_{v}S_{v}\left(t\right), \end{array}$$

and its solution is given by

(56) $$\begin{array}{c} S_{v}\left(t\right)=\frac{\Pi }{\mu_{v}}+S_{v,0}e^{-\mu_{v}t}-R_{v,0}e^{-\left(\rho +\mu_{v}\right)t}. \end{array}$$

Now, suppose that the time, *t*⟶∞, we need to show that *X*⟶*X*^∗^. Obviously, *R*_*h*_(*t*)⟶0, *R*_*v*_(*t*)⟶0 as *t*⟶∞. Thus, *S*_*h*_(*t*)⟶*Λ*/*μ*, *S*_*v*_(*t*)⟶*Π*/*μ*_*v*_ as *t*⟶∞, regardless of the values of *S*_*h*_(0), *R*_*h*_(0) and *S*_*v*_(0), *R*_*v*_(0), respectively. Thus, all points with respect to this condition converge at *X*_0_^∗^ = (*Λ*/*μ*, 0, *Π*/*μ*_*v*_, 0). Hence, *X*^∗^ = (*Λ*/*μ*, 0, *Π*/*μ*_*v*_, 0) is GAS.

The article "A Mathematical Model Analysis for the Transmission Dynamics of Leptospirosis Disease in Human and Rodent Populations" was published in 2022. Journal: Comput Math Methods Med.

Next, we have

(57) $$\begin{array}{c} G\left(X,Y\right)=\left[\begin{array}{c} G_{1}\left(X,Y\right)\\ G_{2}\left(X,Y\right)\\ G_{3}\left(X,Y\right)\\ G_{4}\left(X,Y\right) \end{array}\right]=\left[\begin{array}{c} \left(\frac{\beta_{2}B_{l}}{\kappa +B_{l}}+\beta_{1}I_{v}\right)S_{h}-\left(\theta +\mu \right)E_{h}\\ \theta E_{h}-\left(\alpha +\delta +\mu \right)I_{h}\\ \beta_{3}S_{v}I_{h}-\left(\sigma +\mu_{v}\right)I_{v}\\ \tau_{1}I_{h}+\tau_{2}I_{v}-\mu_{b}B_{l} \end{array}\right]. \end{array}$$

We can then obtain

(58) $$\begin{array}{c} A=\frac{\partial G\left(X^{*},0\right)}{\partial Y}=\left[\begin{array}{cccc} -\left(\theta +\mu \right) & 0 & \frac{\beta_{1}\Lambda }{\mu } & \frac{\beta_{2}\Lambda }{\kappa \mu }\\ \theta & -\left(\alpha +\delta +\mu \right) & 0 & 0\\ 0 & \frac{\beta_{3}\Pi }{\mu_{v}} & -\left(\sigma +\mu_{v}\right) & 0\\ 0 & \tau_{1} & \tau_{2} & -\mu_{b} \end{array}\right], \end{array}$$

which is clearly an *M*-matrix

(59) $$\begin{array}{c} G^{⋆}\left(X,Y\right)=AY-G\left(X,Y\right)=\left[\begin{array}{c} \beta_{1}I_{v}\left(\frac{\Lambda }{\mu }-S_{h}\right)+\frac{\beta_{2}B_{l}}{\kappa }\left(\frac{\Lambda }{\mu }-\frac{\kappa S_{h}}{\kappa +B_{l}}\right)\\ 0\\ \beta_{3}I_{h}\left(\frac{\Pi }{\mu_{v}}-S_{v}\right)\\ 0 \end{array}\right]. \end{array}$$

Since all parameters are nonnegative, 0 ≤ (*κS*_*h*_/(*κ* + *B*_*l*_)) ≤ *S*_*h*_ ≤ *Λ*/*μ*(∵(*κ*/(*κ* + *B*_*l*_)) ≤ 1), 0 ≤ *S*_*v*_ ≤ *Π*/*μ*_*v*_. It follows that (*Λ*/*μ* − *S*_*h*_) ≥ 0, ((*Λ*/*μ*) − (*κS*_*h*_/(*κ* + *B*_*l*_))) ≥ 0, and (*Π*/*μ*_*v*_ − *S*_*v*_) ≥ 0.

The article "A Mathematical Model Analysis for the Transmission Dynamics of Leptospirosis Disease in Human and Rodent Populations" was published in 2022. Journal: Comput Math Methods Med.

Hence, *G*^⋆^(*X*, *Y*) ≥ 0∀ (*X*, *Y*) ∈ Γ. Therefore, the disease-free equilibrium point, *ε*_0*l*_^∗^ = (*Λ*/*μ*, 0, 0, 0, *Π*/*μ*_*v*_, 0, 0, 0), of the model (3) is globally asymptotically stable. This completes the proof.

**Remark 1 .**

The model (3) does not exhibit a backward bifurcation at *R*_0_ = 1 when *R*_0_ < 1, since DFE is the only stable (or positive) equilibrium point for *R*_0_ < 1 in the Theorem 4.

The backward bifurcation has been observed in the leptospirosis epidemic model [16].

### 3.6. Endemic Equilibrium (EE)

The EE point of our model is computed by setting the system of differential equations in (3) to zero. Thus, it is obtained by *dS*_*h*_^∗^/*dt* = *dE*_*h*_^∗^/*dt* = *dI*_*h*_^∗^/*dt* = *dR*_*h*_^∗^/*dt* = *dS*_*v*_^∗^/*dt* = *dI*_*v*_^∗^/*dt* = *dR*_*v*_^∗^/*dt* = *dB*_*l*_^∗^/*dt* = 0, which is given by *E*_*l*_^∗^ = (*S*_*h*_^∗^, *E*_*h*_^∗^, *I*_*h*_^∗^, *R*_*h*_^∗^, *S*_*v*_^∗^, *I*_*v*_^∗^, *R*_*v*_^∗^, *B*_*l*_^∗^), where all disease states are considered to be positive, and thus, *I*_*h*_^∗^ must be greater than zero for all the other states to be positive. Now, by setting the system of equations in (3) to zero at steady state, we have

(60) $$\begin{array}{c} \left\{\begin{array}{c} \frac{dS_{h}^{*}}{dt}=\Lambda +\gamma R_{h}^{*}-\left(\beta_{2}\frac{B_{l}^{*}}{\kappa +B_{l}^{*}}+\beta_{1}I_{v}^{*}+\mu \right)S_{h}^{*}=0,\\ \frac{dE_{h}}{dt}=\left(\beta_{2}\frac{B_{l}^{*}}{\kappa +B_{l}^{*}}+\beta_{1}I_{v}^{*}\right)S_{h}^{*}-\left(\theta +\mu \right)E_{h}^{*}=0,\\ \begin{array}{c} \frac{dI_{h}^{*}}{dt}=\theta E_{h}^{*}-\left(\alpha +\delta +\mu \right)I_{h}^{*}=0,\\ \frac{dR_{h}^{*}}{dt}=\delta I_{h}^{*}-\left(\gamma +\mu \right)R_{h}^{*}=0,\\ \begin{array}{c} \frac{dS_{v}^{*}}{dt}=\Pi +\rho R_{v}^{*}-\left(\beta_{3}I_{h}^{*}+\mu_{v}\right)S_{v}^{*}=0,\\ \frac{dI_{v}^{*}}{dt}=\beta_{3}I_{h}^{*}S_{v}^{*}-\left(\sigma +\mu_{v}\right)I_{v}^{*}=0,\\ \begin{array}{c} \frac{dR_{v}^{*}}{dt}=\sigma I_{v}^{*}-\left(\rho +\mu_{v}\right)R_{v}^{*}=0,\\ \frac{dB_{l}^{*}}{dt}=\tau_{1}I_{h}^{*}+\tau_{2}I_{v}^{*}-\mu_{b}B_{l}^{*}=0. \end{array} \end{array} \end{array} \end{array}\right. \end{array}$$

Due to the complexity of the model system (3), all other state variables at the steady state are expressed in terms of the steady state of *I*_*h*_ which is denoted as *I*_*h*_^∗^. Accordingly, we found as

(61) $$\begin{array}{c} E_{l}^{*}=\left(S_{h}^{*},E_{h}^{*},I_{h}^{*},R_{h}^{*},S_{v}^{*},I_{v}^{*},R_{v}^{*},B_{l}^{*}\right),=\left(\frac{\Lambda +\gamma R_{h}^{*}}{\lambda^{*}+\mu },\frac{\varepsilon_{2}}{\theta }I_{h}^{*},I_{h}^{*},\frac{\delta }{\varepsilon_{3}}I_{h}^{*},\frac{\Pi +\rho R_{v}^{*}}{\beta_{3}I_{h}^{*}+\mu_{v}},\frac{\beta_{3}\Pi \varepsilon_{5}I_{h}^{*}}{\mu_{v}\left(\varepsilon_{4}\varepsilon_{5}+\beta_{3}\varepsilon_{6}I_{h}^{*}\right)},\frac{\beta_{3}\Pi \sigma I_{h}^{*}}{\mu_{v}\left(\varepsilon_{4}\varepsilon_{5}+\beta_{3}\varepsilon_{6}I_{h}^{*}\right)},\frac{\tau_{1}I_{h}^{*}+\tau_{2}I_{v}^{*}}{\mu_{b}}\right), \end{array}$$

where

(62) $$\begin{array}{c} \varepsilon_{1}=\theta +\mu ,\\ \varepsilon_{2}=\alpha +\delta +\mu ,\\ \varepsilon_{3}=\gamma +\mu ,\\ \varepsilon_{4}=\sigma +\mu_{v},\\ \varepsilon_{5}=\rho +\mu_{v},\\ \varepsilon_{6}=\sigma +\rho +\mu_{v}. \end{array}$$

By combining the equations of (61) and the first and second equations of the model system (3), we obtained a septic (or heptic) polynomial equation for *I*_*h*_^∗^ which is described as follows:

(63) $$\begin{array}{c} P\left(I_{h}^{*}\right)=I_{h}^{*}\left(A{\left(I_{h}^{*}\right)}^{6}+B{\left(I_{h}^{*}\right)}^{5}+C{\left(I_{h}^{*}\right)}^{4}+D{\left(I_{h}^{*}\right)}^{3}+E{\left(I_{h}^{*}\right)}^{2}+FI_{h}^{*}+G\right)=0, \end{array}$$

where

(64) $$\begin{array}{c} A=-\left[\Psi_{3}\Psi_{7}\eta_{4}+\Psi_{7}^{2}\left(\theta +\mu \right)\left(\alpha +\delta +\mu \right)\left(\gamma +\mu \right)\mu \right]<0\text{ always},\\ B=-\eta_{4}\left(\Psi_{2}\Psi_{7}+\Psi_{3}\Psi_{6}\right)+\Psi_{7}\eta_{3}\left(\theta +\mu \right)\left(\alpha +\delta +\mu \right)\left(\gamma +\mu \right)\left.\mu \right)\left[\eta_{3}^{2}\kappa \mu_{b}\left(R_{b}-1\right)+\eta_{3}\tau_{1}\left(\sigma +\mu_{v}\right)\left(\rho +\mu_{v}\right)\mu_{v}\left(R_{v}-1\right)-\eta_{3}\left(\eta_{2}\tau_{1}+\eta_{1}\tau_{2}\right)-\Psi_{6}\right]<0\text{ if }R_{0}<1,\\ C=-\eta_{4}\left(\Psi_{1}\Psi_{7}+\Psi_{2}\Psi_{6}+\Psi_{3}\Psi_{5}\right)+\Psi_{7}\Omega_{2}-\Psi_{7}\Psi_{5}\left(\theta +\mu \right)\left(\alpha +\delta +\mu \right)\left(\gamma +\mu \right)\mu +\Psi_{6}\Omega_{3}=-\eta_{4}\left(\Psi_{1}\Psi_{7}+\Psi_{2}\Psi_{6}+\Psi_{3}\Psi_{5}\right)+\Psi_{6}\Omega_{3}+\left(\gamma +\mu \right)\left(\theta +\mu \right)\left(\alpha +\delta +\mu \right)\mu \left[\eta_{2}\eta_{3}\kappa \mu_{b}2\left(R_{b}-1\right)+\left(\sigma +\mu_{v}\right)\left(\rho +\mu_{v}\right)\mu_{v}\left(R_{v}-2\right)\left(\eta_{3}\kappa \mu_{b}+\eta_{2}\tau_{1}+\eta_{1}\tau_{2}\right)\right]<0\text{ if }R_{0}<1,\\ D=-\eta_{4}\left(\Psi_{1}\Psi_{6}+\Psi_{2}\Psi_{5}+\Psi_{3}\Psi_{4}\right)+\Psi_{7}\left[\Omega_{1}-\Psi_{4}\left(\theta +\mu \right)\left(\alpha +\delta +\mu \right)\left(\gamma +\mu \right)\mu \right]+\left.\Psi_{6}\Omega_{2}+\Psi_{5}\Omega_{3}\right),\\ E=-\eta_{4}\left(\Psi_{1}\Psi_{5}+\Psi_{2}\Psi_{4}\right)+\Psi_{6}\Omega_{1}+\Psi_{5}\Omega_{2}+\Psi_{4}\Omega_{3},\\ F=-\eta_{4}\Psi_{1}\Psi_{4}+\Psi_{5}\Omega_{1}+\Psi_{4}\Omega_{2},G=\Psi_{4}\Omega_{1}<0\text{ if }R_{0}<1, \end{array}$$

with

(65) $$\begin{array}{c} \eta_{1}=\Pi \beta_{3}\left(\rho +\mu_{v}\right),\\ \eta_{2}=\mu_{v}\left(\sigma +\mu_{v}\right)\left(\rho +\mu_{v}\right),\\ \eta_{3}=\beta_{3}\mu_{v}\left(\sigma +\rho +\mu_{v}\right),\\ \eta_{4}=\theta \gamma \left(\alpha +\mu \right)+\mu \left(\alpha +\delta +\mu \right)\left(\theta +\gamma +\mu \right),\\ \Psi_{1}=\eta_{2}\left(\beta_{2}\left(\eta_{2}\tau_{1}+\eta_{1}\tau_{2}\right)+\beta_{1}\kappa \eta_{1}\mu_{b}\right),\\ \Psi_{2}=\left(\eta_{2}\tau_{1}+\eta_{1}\tau_{2}\right)\left(\beta_{2}\eta_{3}+\beta_{1}\eta_{1}\right)+\eta_{3}\left(\beta_{2}\eta_{2}\tau_{1}+\beta_{1}\kappa \eta_{1}\mu_{b}\right),\\ \Psi_{3}=\eta_{3}\tau_{1}\left(\beta_{2}\eta_{3}+\beta_{1}\eta_{1}\right),\\ \Psi_{4}=\kappa \eta_{2}^{2}\mu_{b},\\ \Psi_{5}=2\kappa \eta_{2}\eta_{3}\mu_{b}+\eta_{2}\left(\eta_{2}\tau_{1}+\eta_{1}\tau_{2}\right),\\ \Psi_{6}=\eta_{3}\left(\kappa \eta_{3}\mu_{b}+2\eta_{2}\tau_{1}+\eta_{1}\tau_{2}\right),\\ \Psi_{7}=\eta_{3}^{2}\tau_{1},\\ \Omega_{1}=\left(\gamma +\mu \right)\left[\Psi_{1}\Lambda \theta -\Psi_{4}\left(\theta +\mu \right)\left(\alpha +\delta +\mu \right)\mu \right]=\eta_{2}\kappa \mu_{b}\mu_{v}\mu \left(\theta +\mu \right)\left(\alpha +\delta +\mu \right)\left(\gamma +\mu \right)\left(\sigma +\mu_{v}\right)\left(\rho +\mu_{v}\right)\left(R_{0}-1\right)\left(R_{0}-R_{b}+1\right),\\ \Omega_{2}=\left(\gamma +\mu \right)\left[\Psi_{2}\Lambda \theta -\Psi_{5}\left(\theta +\mu \right)\left(\alpha +\delta +\mu \right)\mu \right]=\left(\gamma +\mu \right)\left(\theta +\mu \right)\left(\alpha +\delta +\mu \right)\mu \left[\eta_{2}\eta_{3}\kappa \mu_{b}\left(2R_{b}-1\right)+\left(\sigma +\mu_{v}\right)\left(\rho +\mu_{v}\right)\mu_{v}\left(R_{v}-1\right)\left(\eta_{3}\kappa \mu_{b}+\eta_{2}\tau_{1}+\eta_{1}\tau_{2}\right)\right],\\ \Omega_{3}=\left(\gamma +\mu \right)\left[\Psi_{3}\Lambda \theta -\Psi_{6}\left(\theta +\mu \right)\left(\alpha +\delta +\mu \right)\mu \right]=\eta_{3}\left(\theta +\mu \right)\left(\alpha +\delta +\mu \right)\mu \left[\eta_{3}^{2}\kappa \mu_{b}\left(R_{b}-1\right)+\eta_{3}\tau_{1}\left(\sigma +\mu_{v}\right)\left(\rho +\mu_{v}\right)\mu_{v}\left(R_{v}-1\right)-\left(\eta_{2}\tau_{1}+\eta_{1}\tau_{2}\right)\right). \end{array}$$

The article "A Mathematical Model Analysis for the Transmission Dynamics of Leptospirosis Disease in Human and Rodent Populations" was published in 2022. Journal: Comput Math Methods Med.

### 3.7. Local Stability of the Endemic Equilibrium

**Theorem 5 .**

The endemic equilibrium *E*_*l*_^∗^ of the model (3) is locally asymptotically stable for *R*_0_ > 1 (but near 1) (based on Theorem 4.1 by [24]).

**Proof**

Now, consider the system of equations (3). To investigate the nature of the bifurcation, we use the method introduced in Theorem 4.1 by [24]. To apply this method, the following simplification and change of variables are made first of all. Let *S*_*h*_ = *x*_1_, *E*_*h*_ = *x*_2_, *I*_*h*_ = *x*_3_, *R*_*h*_ = *x*_4_, *S*_*v*_ = *x*_5_, *I*_*v*_ = *x*_6_, *R*_*v*_ = *x*_7_, and *B*_*l*_ = *x*_8_.

By using vector notation,

(66) $$\begin{array}{c} X={\left(x_{1},x_{2},x_{3},x_{4},x_{5},x_{6},x_{7},x_{8}\right)}^{T}. \end{array}$$

The model system (3) can be written as

(67) $$\begin{array}{c} \frac{dX}{dt}=F\left(X\right), \end{array}$$

where *F* = (*f*_1_, *f*_2_, *f*_3_, *f*_4_, *f*_5_, *f*_6_, *f*_7_, *f*_8_)^*T*^.

The following system of differential equations is established:

(68) $$\begin{array}{c} \left\{\begin{array}{c} \frac{dx_{1}}{dt}=\Lambda +\gamma x_{4}-\left(\frac{\beta_{2}x_{8}}{\kappa +x_{8}}+\beta_{1}x_{6}+\mu \right)x_{1}=f_{1},\\ \frac{dx_{2}}{dt}=\left(\frac{\beta_{2}x_{8}}{\kappa +x_{8}}+\beta_{1}x_{6}+\mu \right)x_{1}-\left(\theta +\mu \right)x_{2}=f_{2},\\ \begin{array}{c} \frac{dx_{3}}{dt}=\theta x_{2}-\left(\alpha +\delta +\mu \right)x_{3}=f_{3},\\ \frac{dx_{4}}{dt}=\delta x_{3}-\left(\gamma +\mu \right)x_{4}=f_{4},\\ \begin{array}{c} \frac{x_{5}}{dt}=\Pi +\rho x_{7}-\left(\beta_{3}x_{3}+\mu_{v}\right)x_{5}=f_{5},\\ \frac{dx_{6}}{dt}=\beta_{3}x_{3}x_{5}-\left(\sigma +\mu_{v}\right)x_{6}=f_{6},\\ \begin{array}{c} \frac{dx_{7}}{dt}=\sigma x_{6}-\left(\rho +\mu_{v}\right)x_{7}=f_{7},\\ \frac{dx_{8}}{dt}=\tau_{1}x_{3}+\tau_{2}x_{6}-\mu_{b}x_{8}=f_{8}. \end{array} \end{array} \end{array} \end{array}\right. \end{array}$$

Choosing *β*_1_^∗^ as bifurcation parameter and solving for *β*_1_^∗^ from equation (37) when *R*_0_ = 1, we obtained as

(69) $$\begin{array}{c} \beta_{1}^{*}=\frac{\kappa \mu \mu_{b}\mu_{v}\varepsilon_{1}\varepsilon_{2}\varepsilon_{4}-\beta_{3}\Pi \Lambda \theta \left(\tau_{1}\kappa \mu_{b}+\beta_{2}\Pi \tau_{2}\right)}{\beta_{3}\Pi \Lambda \theta \kappa \mu_{b}}. \end{array}$$

Considering *β*_1_ = *β*_1_^∗^, the Jacobian of the system (68) evaluated at (*ε*_0_^∗^*l*, *β*_1_^∗^) is given by

(70) Jε0l∗,β1∗=−μ00γ0−J10−J20−J3000J10J20θ−J40000000δ−J50000 0−J60−μv0ρ000−J600−J70000000σ0000τ100τ20−μb,

where *J*_1_ = *β*_1_^∗^*Λ*/*μ*, *J*_2_ = *β*_2_*Λ*/*κμ*, *J*_3_ = *θ* + *μ*, *J*_4_ = *α* + *δ* + *μ*, *J*_5_ = *γ* + *μ*, *J*_6_ = *β*_3_*Π*/*μ*_*v*_, *J*_7_ = *σ* + *μ*_*v*_, and *J*_8_ = *ρ* + *μ*_*v*_.

The characteristic polynomial equation of the matrix *J*(*ε*_0*l*_^∗^, *β*_1_^∗^) is given by

(71) $$\begin{array}{c} P^{*}\left(\lambda \right)=\lambda \left(\lambda +\mu \right)\left(\lambda +\mu_{v}\right)\left(\lambda +\gamma +\mu \right)\left(\lambda +\rho +\mu_{v}\right)\left[\lambda^{3}+A_{1}\lambda^{2}+A_{2}\lambda +A_{3}\right]=0, \end{array}$$

where

(72) $$\begin{array}{c} A_{1}=\left(\theta +\mu \right)+\left(\alpha +\delta +\mu \right)+\left(\sigma +\mu_{v}\right)+\mu_{b},\\ A_{2}=\left(\theta +\mu \right)\left(\mu_{b}+\alpha +\delta +\mu +\sigma +\mu_{v}\right)+\mu_{b}\left(\alpha +\delta +\mu +\sigma +\mu_{v}\right)+\left(\alpha +\delta +\mu \right)\left(\sigma +\mu_{v}\right),\\ A_{3}=J_{7}\mu_{b}\left(J_{3}+J_{4}\right)+J_{3}J_{4}\mu_{b}\left(1-R_{b}\right)+J_{3}J_{4}J_{7}\left(1-R_{v}\right),=\left(\sigma +\mu_{v}\right)\mu_{b}\left(\theta +2\mu +\alpha +\delta \right)+\left(\theta +\mu \right)\left(\alpha +\delta +\mu \right)\mu_{b}Rv+\left(\theta +\mu \right)\left(\alpha +\delta +\mu \right)\left(\sigma +\mu_{v}\right)\mu_{b}R_{b}. \end{array}$$

Thus, *λ*_1_ = 0, *λ*_2_ = −*μ*, *λ*_3_ = −*μ*_*v*_, *λ*_4_ = −(*γ* + *μ*), and *λ*_5_ = −(*ρ* + *μ*_*v*_) are the five eigenvalues of *J*(*ε*_0*l*_^∗^, *β*_1_^∗^). The remaining three eigenvalues are the zeros of the polynomial equation *λ*^3^ + *A*_1_*λ*^2^ + *A*_2_*λ* + *A*_3_ = 0, since *A*_1_ > 0, *A*_2_ > 0, *A*_3_ > 0, *A*_1_*A*_2_ − *A*_3_ > 0 for *R*_0_ = 1 (see the proof of theorem (3.3.3)). We conclude that zero is a simple eigenvalue of *J*(*ε*_0*l*_^∗^, *β*_1_^∗^) and all other eigenvalues of *J*(*ε*_0_^∗^*l*, *β*_1_^∗^) have negative real numbers or real parts. This is an indication that the center manifold theorem is applicable. We first compute the left and right eigenvectors of the Jacobian matrix *J*(*ε*_0_^∗^*l*, *β*_1_^∗^). let *Y* = (*y*_1_, *y*_2_, *y*_3_, *y*_4_, *y*_5_, *y*_6_, *y*_7_, *y*_8_)^*T*^ be the right eigenvector of *J*(*ε*_0_^∗^*l*, *β*_1_^∗^) corresponding to *λ* = 0. Then, *Y* is computed as

(73) −μ00γ0−J10−J20−J3000J10J20θ−J40000000δ−J50000 0−J60−μv0ρ000−J600−J70000000σ0000τ100τ20−μby1y2y3y4y5y6y7y8=00000000.

The article "A Mathematical Model Analysis for the Transmission Dynamics of Leptospirosis Disease in Human and Rodent Populations" was published in 2022. Journal: Comput Math Methods Med.

Then, equation (73) can be expressed as

(74) $$\begin{array}{c} -\mu y_{1}-\gamma y_{4}-J_{1}y_{6}-J_{2}y_{8}=0,\\ -J_{6}y_{3}-\mu_{v}y_{5}+\rho y_{7}=0,\\ -J_{3}y_{2}+J_{1}y_{6}+J_{2}y_{8}=0,\\ J_{6}y_{3}-J_{7}y_{6}=0,\\ \theta y_{2}-J_{4}y_{3}=0,\\ \rho y_{6}-J_{8}y_{7}=0,\\ \delta y_{3}-J_{5}y_{4}=0,\\ \tau_{1}y_{3}+\tau_{2}y_{6}-\mu_{b}y_{8}=0. \end{array}$$

The components of *Y* can be obtained from (74) as

(75) $$\begin{array}{c} \left\{\begin{array}{c} y_{1}=-y_{3}\frac{\left[\theta \gamma \left(\alpha +\mu \right)+\mu \left(\alpha +\delta +\mu \right)\left(\theta +\gamma +\mu \right.\right]}{\theta \mu \left(\gamma +\mu \right)}<0,\\ y_{2}=y_{3}\left(\frac{\alpha +\delta +\mu }{\theta }\right)>0,\\ \begin{array}{c} y_{3}=y_{3}>0,\\ y_{4}=y_{3}\left(\frac{\delta }{\gamma +\mu }\right)>0,\\ \begin{array}{c} y_{5}=y_{3}\left(\frac{\beta_{3}\Pi \mu_{v}\left(\sigma +\rho +\mu_{v}\right)}{\mu_{v}\left(\sigma +\mu_{v}\right)\left(\rho +\mu_{v}\right)}\right)>0,\\ y_{6}=y_{3}\left(\frac{\beta_{3}\Pi }{\mu_{v}\left(\sigma +\mu_{v}\right)}\right)>0,\\ \begin{array}{c} y_{7}=y_{3}\left(\frac{\beta_{3}\Pi \sigma }{\mu_{v}\left(\sigma +\mu_{v}\right)\left(\rho +\mu_{v}\right)}\right)>0,\\ y_{8}=y_{3}\left(\frac{\mu_{v}\tau_{1}\left(\sigma +\mu_{v}\right)+\beta_{3}\Pi \left(\sigma +\mu_{v}\right)\tau_{2}}{\mu_{v}\mu_{b}\left(\sigma +\mu_{v}\right)}\right)>0. \end{array} \end{array} \end{array} \end{array}\right. \end{array}$$

Next, the left eigenvector *Z* = (*z*_1_, *z*_2_, *z*_3_, *z*_4_, *z*_5_, *z*_6_, *z*_7_, *z*_8_)^*T*^ of the Jacobian matrix *J*(*ε*_0_^∗^*l*, *β*_1_^∗^) corresponding to *λ* = 0 is computed as

(76) −μ00000000−J3θ0000000−J4δ−J6J60τ1γ00−J500000000−μv000−J1J1000−J4στ20000ρ0−J80−J2J200000−μb        z1z2z3z4z5z6z7z8=00000000.

Thus, *Z* can be found as

(77) $$\begin{array}{c} Z=\left(0,z_{2},z_{2}\frac{\left(\theta +\mu \right)}{\theta },0,0,z_{2}\frac{\mu_{v}\left(\mu \mu_{b}\kappa \left(\theta +\mu \right)\left(\alpha +\delta +\mu \right)-\beta_{2}\Lambda \theta \tau_{1}\right)}{\beta_{3}\Pi \mu \mu_{b}\kappa \theta },0,z_{2}\frac{\beta_{2}\Lambda }{\mu \kappa }\right), \end{array}$$

where *z*_2_ > 0 and it is calculated to ensure that the eigenvectors satisfy the condition *Z*. *Y* = 1, for *R*_0_ = 1.

The local stability near the bifurcation point *β*_1_ = *β*_1_^∗^ is determined by the signs of two associated constants *a* and *b*. Based on the center manifold theorem 4.1 in [24], we compute the coefficients *a* and *b*, as

(78) $$\begin{array}{c} a=\overset{n}{\underset{k,i,j=1}{\sum }}z_{k}y_{i}y_{j}\frac{\partial^{2}f_{k}}{\partial x_{i}\partial x_{j}}\left(\varepsilon_{0l}^{*},\beta_{1}^{*}\right),\\ b=\overset{n}{\underset{k,i=1}{\sum }}z_{k}y_{i}\frac{\partial^{2}f_{k}}{\partial x_{i}\beta_{1}^{*}}\left(\varepsilon_{0l}^{*},\beta_{1}^{*}\right). \end{array}$$

Since the first, fourth, fifth, and seventh components of *Z* are zero, we do not need the derivatives of *f*_1_, *f*_4_, *f*_5_, and *f*_7_. The derivatives of *f*_2_, *f*_3_, *f*_6_, and *f*_8_ are *∂*^2^*f*_2_/*∂x*_1_*∂x*_6_ = *∂*^2^*f*_2_/*∂x*_6_*∂x*_1_ = *β*_1_, *∂*^2^*f*_2_/*∂x*_1_*∂x*_8_ = *∂*^2^*f*_2_/*∂x*_8_*∂x*_1_ = *β*_2_/*κ*, (*∂*^2^*f*_2_/*∂x*_6_*∂β*_1_^∗^)(*ε*_0*l*_^∗^, *β*_1_^∗^) = *Λ*/*μ*, and (*∂*^2^*f*_2_/*∂x*_8_^2^)(*ε*_0*l*_^∗^, *β*_1_^∗^) = −2*β*_2_*Λ*/*κ*^2^*μ*, and any other second order partial derivative of *f*_*k*_ is zero, ∀*k* = 1, 2, 3, 4, 5, 6, 7, 8.

It follows that

(79) $$\begin{array}{c} a=\overset{n}{\underset{k,i,j=1}{\sum }}z_{k}y_{i}y_{j}\frac{\partial^{2}f_{k}}{\partial x_{i}\partial x_{j}}\left(\varepsilon_{0l}^{*},\beta_{1}^{*}\right)=z_{2}y_{1}y_{6}\frac{\partial^{2}f_{2}}{\partial x_{1}\partial x_{6}}\left(\varepsilon_{0l}^{*},\beta_{1}^{*}\right)+z_{2}y_{1}y_{8}\frac{\partial^{2}f_{2}}{\partial x_{1}\partial x_{8}}\left(\varepsilon_{0l}^{*},\beta_{1}^{*}\right)+z_{2}y_{8}^{2}\frac{\partial^{2}f_{2}}{\partial x_{8}^{2}}\left(\varepsilon_{0l}^{*},\beta_{1}^{*}\right). \end{array}$$

Substituting the values for partial derivatives and *y*_1_, *y*_8_, we obtain

(80) $$\begin{array}{c} a=-z_{2}y_{3}^{2}\left[\beta_{3}\beta_{1}\Pi \sigma \Phi +\frac{\beta_{2}\Phi \left[\mu_{v}\tau_{1}\left(\sigma +\mu_{v}\right)+\beta_{3}\Pi \tau_{2}\right]}{\kappa \mu_{b}}+\frac{\beta_{2}\Lambda }{\kappa^{2}\mu }{\left(\frac{\mu_{v}\tau_{1}\left(\sigma +\mu_{v}\right)+\beta_{3}\Pi \tau_{2}}{\mu_{v}\mu_{b}\left(\sigma +\mu_{v}\right)}\right)}^{2}\right]<0. \end{array}$$

where *Φ* = [*θγ*(*α* + *μ*) + *μ*(*α* + *δ* + *μ*)(*θ* + *γ* + *μ*)]/*θμ*_*v*_*μ*(*γ* + *μ*)(*σ* + *μ*_*v*_) and

(81) $$\begin{array}{c} b=z_{2}y_{6}\frac{\partial^{2}f_{2}}{\partial x_{6}\partial \beta_{1}^{*}}\left(\varepsilon_{0l}^{*},\beta_{1}^{*}\right)=z_{2}y_{3}\left(\frac{\beta_{3}\Pi \Lambda }{\mu_{v}\mu \left(\sigma +\mu_{v}\right)}\right)>0\left(\text{always}\right). \end{array}$$

Since *a* <0 and *b* >0 and with the help of Theorem 4.1 by Castillo-Chavez and Song in [24], it is confirmed that the system follows a forward bifurcation at *R*_0_ = 1 (see Figure 2), and hence, the endemic equilibrium is locally asymptotically stable for *R*_0_ > 1, but sufficiently close to 1

The epidemiological implication of this shows that the leptospirosis disease can be eradicated in infected population as long as when *R*_0_ < 1. The condition *R*_0_ < 1 is necessary and sufficient for disease elimination for a model that undergoes the forward bifurcation [25].

The article "A Mathematical Model Analysis for the Transmission Dynamics of Leptospirosis Disease in Human and Rodent Populations" was published in 2022. Journal: Comput Math Methods Med.

## 4. Sensitivity Analysis

In this section, we investigated the sensitivity of the parameters for the basic reproduction of the model using the idea presented in [26–28]. It is important to carry out the sensitivity of the basic reproduction number *R*_0_ for its parameters. This will give parameters with a high impact on the leptospirosis model (3) and therefore allow to target on control measures to reduce the transmission of the disease. To measure the sensitivity index of *R*_0_ to a given parameter *β*, we use the following relation:

(82) $$\begin{array}{c} \Omega_{\beta }^{R_{0}}=\left(\frac{\partial R_{0}}{\partial \beta }\right)\left(\frac{\beta }{R_{0}}\right). \end{array}$$

An analytical expression for the sensitivity index of each parameter involved in *R*_0_ is derived as follows:

(83) $$\begin{array}{c} \Omega_{\beta_{1}}^{R_{0}}=\frac{R_{v}}{R_{0}\left(2R_{0}-R_{b}\right)}>0\left(∵R_{0}>R_{b}\right),\\ \Omega_{\beta_{2}}^{R_{0}}=\frac{R_{b}\left(2R_{0}-R_{b}\right)+R_{b}^{2}+2R_{v}}{2R_{0}\left(2R_{0}-R_{b}\right)}>0,\\ \Omega_{\Lambda }^{R_{0}}=\frac{R_{b}\left(2R_{0}-R_{b}\right)+R_{b}^{2}+2R_{hv}}{2R_{0}\left(2R_{0}-R_{b}\right)}>0,\\ \Omega_{\Pi }^{R_{0}}=\frac{R_{hv}}{R_{0}\left(2R_{0}-R_{b}\right)}>0,\\ \Omega_{\mu }^{R_{0}}=-\left(\frac{\left[R_{b}\left(2R_{0}-R_{b}\right)+R_{b}^{2}+2R_{hv}\right]\left[\varepsilon_{1}\varepsilon_{2}+\mu \left(\varepsilon_{1}+\varepsilon_{2}\right)\right]}{2R_{0}\left(2R_{0}-R_{b}\right)}\right)<0,\\ \Omega_{\beta_{3}}^{R_{0}}=\frac{R_{hv}}{R_{0}\left(2R_{0}-R_{b}\right)}>0,\\ \Omega_{\theta }^{R_{0}}=\frac{\mu \left[R_{b}\left(2R_{0}-R_{b}\right)+R_{b}^{2}+2R_{hv}\right]}{2R_{0}\left(2R_{0}-R_{b}\right)}>0,\\ \Omega_{\mu_{v}}^{R_{0}}=-\frac{\left(\varepsilon_{4}+\mu_{v}\right)R_{hv}}{R_{0}\left(2R_{0}-R_{b}\right)}<0,\\ \Omega_{\alpha }^{R_{0}}=-\frac{\alpha }{\varepsilon_{2}}\left(\frac{R_{b}\left(2R_{0}-R_{b}\right)+R_{b}^{2}+2R_{hv}}{2R_{0}\left(2R_{0}-R_{b}\right)}\right)<0,\\ \Omega_{\tau_{1}}^{R_{0}}=\frac{R_{b}\left(2R_{0}-R_{b}\right)+R_{b}^{2}}{2R_{0}\left(2R_{0}-R_{b}\right)}>0,\\ \Omega_{\delta }^{R_{0}}=-\frac{\delta }{\varepsilon_{2}}\left(\frac{R_{b}\left(2R_{0}-R_{b}\right)+R_{b}^{2}+2R_{hv}}{2R_{0}\left(2R_{0}-R_{b}\right)}\right)<0,\\ \Omega_{\sigma }^{R_{0}}=-\left(\frac{\sigma R_{hv}}{\varepsilon_{4}R_{0}\left(2R_{0}-R_{b}\right)}\right)<0,\\ \Omega_{\tau_{2}}^{R_{0}}=\frac{R_{h}}{R_{0}\left(2R_{0}-R_{b}\right)}>0,\\ \Omega_{\kappa }^{R_{0}}=-\frac{R_{b}R_{0}+R_{h}}{R_{0}\left(2R_{0}-R_{b}\right)}<0,\\ \Omega_{\mu_{b}}^{R_{0}}=-\frac{R_{b}R_{0}+R_{h}}{R_{0}\left(2R_{0}-R_{b}\right)}<0. \end{array}$$

The values of the sensitivity indices of *R*_0_ to each of its parameter values are computed and listed in Table 3 in decreasing order of sensitivity indices from the most to the least sensitive parameter. We used an algorithm Markov Chain Monte Carlo (MCMC) to fit parameter values of the model. The parameter values were used from previously published papers, and others were estimated as shown in Table 3.

The negative and positive signs of sensitivity index values in Table 3 represent the negative and positive (respectively) influence of parameters on *R*_0_. Thus, from the table, it can be observed that *R*_0_ increases when the values of *Λ*, *Π*, *β*_1_, *β*_2_, *β*_3_, *θ*, *τ*_1_, *τ*_2_are increase and vice versa. On the other hand, increasing the values of *μ*, *μ*_*v*_, *μ*_*b*_, *σ*, *δ*, *α*, *κ* decreases *R*_0_ and vice versa. From the results of sensitivity analysis, the parameters *Λ*, *Π*, *β*_1_, *β*_3_, *μ*, *μ*_*v*_, *δ* are the most influencing on *R*_0_. Further, deceasing *Λ* by 10% decreases *R*_0_ by 5.54%. Increasing *Π* or *β*_3_ by 10% increases *R*_0_ by 4.47%. In contrast, increasing *δ* by 10% decreases *R*_0_ by 3.2%. Similarly, decreasing (or increasing) *μ* and *μ*_*v*_ by a given percentage increases (or decreases, respectively) *R*_0_ by half of the percentage. Epidemiological implications of this is that preventive and control efforts should be targeted on parameters *Λ*, *Π*, *β*_1_, *β*_3_, *μ*_*v*_, *δ* to reduce the burden of the disease in infected population since it is not reasonable biologically or ethically to use the mortality rate of humans as a control measure. In particular, reducing the total number of rodent population can minimize the transmission of disease, since *μ*_*v*_ is the reduction rate of rodents and it has a highly negative influence on *R*_0_. Further, the effect of the most sensitive parameters on disease dynamics behavior is illustrated graphically in the next section.

The article "A Mathematical Model Analysis for the Transmission Dynamics of Leptospirosis Disease in Human and Rodent Populations" was published in 2022. Journal: Comput Math Methods Med.

## 5. Numerical Simulations and Discussions

In this section, we perform some numerical results for the leptospirosis model (3) to demonstrate the results of the qualitative analysis of the model that has been already performed in the previous sections. To do this, we used the fourth-order Runge-Kutta method in the MATLAB program. The parameter values used in the simulations are given in Table 4. These parameter values have taken from previously published papers, and others are estimated as shown in Table 4.

The initial conditions are chosen as (*S*_*h*_(0), *E*_*h*_(0), *I*_*h*_(0), *R*_*h*_(0), *S*_*v*_(0), *I*_*v*_(0), *R*_*v*_(0), *B*_*m*_(0)) = (270,20,10,0, 510,10,0, 100). Using equation (63), parameter values of the Table 4 and the initial conditions, we found that *R*_0_ ≈ 2.8552 > 1, a unique positive endemic equilibrium which given by *E*_*l*_^∗^ = (*S*_*h*_^∗^, *E*_*h*_^∗^, *I*_*h*_^∗^, *R*_*h*_^∗^, *S*_*v*_^∗^, *I*_*v*_^∗^, *R*_*v*_^∗^, *B*_*l*_^∗^) ≈ (47.668,6.5229,5.3154,4.2571,628.6425,34.9632,26.0494,146.2314) with unique positive value *I*_*h*_^∗^ ≈ 5.3154; the other six roots of the polynomial equation (63) are obtained as *I*_0_ = 0, *I*_1_ ≈ −9658.1994, *I*_2_ ≈ −6509.1639, *I*_3_ ≈ −54.7671, *I*_4_≈−47.8513, *I*_5_≈−47.2545.

From graphical illustration of stability analysis of EE, we observed that all trajectories of the model solutions eventually move towards the steady-state *E*_*l*_^∗^ as shown the in Figures 3(a)–3(i) since *E*_*l*_^∗^ the unique positive EE is locally asymptotically stable for *R*_0_ > 1. This shows that the disease persists in population because *R*_0_ = 2.8552 > 1. On the other hand, if changing the values of *β*_1_, *β*_2_, *β*_3_, *μ*_*v*_, and *δ* into 0.0001, 0.0515, 0.0003, 0.0035, and 0.092, respectively, then it yields *R*_0_ ≈ 0.932 < 1. In this case, the model has the DFE which is globally asymptotically stable, and hence, *E*_*l*_^∗^ is unstable. Thus, all trajectories of the model solutions tend to the DFE over time as shown in Figures 4(a)–4(f). Biologically, the implication is that the disease will die out from the community over time, while the susceptible humans and susceptible rodents eventually approach their maximum value for this particular study. Therefore, we should reduce the value of *R*_0_ as much as possible to eradicate the disease rapidly.

The article "A Mathematical Model Analysis for the Transmission Dynamics of Leptospirosis Disease in Human and Rodent Populations" was published in 2022. Journal: Comput Math Methods Med.

### 5.1. Effect of the Transmission Rates of Humans and Rodents (*β*_1_ and *β*_3_) on Dynamics Behavior of the Disease

The transmission rates *β*_1_ and *β*_3_ play a significant role on expansion of the disease transmission by increasing the incidence rates of humans and rodents in the infected population. In this section, we illustrate the sensitivity of the model (3) in human, rodent, and bacterial populations using different values of the parameters. In Figures 5(a) and 5(b), it can be seen that decreasing the human transmission rate (*β*_1_) increases the sizes of susceptible humans and susceptible rodents (eventually) and vice versa. On the other hand, reducing this parameter reduces the sizes of infected individuals, infected rodents, recovered rodents, and bacterial population from the beginning and eventually as shown Figures 5(c)–5(f), respectively. This was performed by taking the values of *β*_1_ as *β*_1_ = 0.00017, *β*_1_ = 0.00023, *β*_1_ = 0.00033, *β*_1_ = 0.0005, and *β*_1_ = 0.0008. In the same manner, we observed the effects for the rodent transmission rate *β*_3_ by setting its values as *β*_3_ = 0.0005, *β*_3_ = 0.0006, *β*_3_ = 0.0007, *β*_3_ = 0.00085, and *β*_3_ = 0.00099 as shown in Figure 6. A decrease (or increase) in the value of human transmission rate *β*_3_ will cause decrease (or increase, respectively) in the size of the infected individuals, infected rodents, and recovered rodents as indicated in Figures 6(b), 6(d), and 6(e), respectively. Similarly, in Figure 6(f), it can be seen that decreasing *β*_3_ decreases the growth bacterial population in an environment with time as they are directly proportional. However, decreasing (or increasing) the human transmission rate (*β*_3_) increases (or decreases, respectively) the size of the number of susceptible humans and susceptible rodents as shown in Figures 6(a) and 6(a), respectively. In view of the simulations of the model in Figures 5 and 6, the smaller parameter values (as possible) will result in the smaller *R*_0_ value and will decrease the incidence rates of human and rodent infections. This shows that reducing the expansion of human infection depends on the reduction of the transmission rates *β*_1_ and *β*_3_ on susceptible individuals and susceptible rodents. Therefore, by minimizing the values of *β*_1_ and *β*_3_ significantly, the number of infected humans, infected rodents, and the growth of leptospires in the environment can be reduced and could finally vanish. This can be achieved by treating infected individuals (using treatment control), avoiding contact with the contaminated environment (soil or water), or by reducing infected rodents as well as the total number of rodent population.

The article "A Mathematical Model Analysis for the Transmission Dynamics of Leptospirosis Disease in Human and Rodent Populations" was published in 2022. Journal: Comput Math Methods Med.

### 5.2. Effect of the Human Recovery Rate (*δ*) on Dynamics Behavior of the Disease

The infectious individuals can be reduced by increasing the value of the human recovery rate (*δ*) using control interventions (treatment of disease infection). In this section, we simulate the model to observe the effect of *δ* in human, rodent, and bacterial populations by varying the value *δ*. From Figure 7, we observed that *δ* is directly proportional with susceptible and recovered individuals as revealed in Figures 7(a) and 7(c). Moreover, it can be seen in Figures 7(b), 7(e), and 7(f) that the population of infected humans and infected rodents and population of bacterial increase (or decrease) from the beginning and eventually as *δ* decreases (or increases, respectively), whereas the size of susceptible rodents increases (or decreases) from the beginning and eventually as *δ* increases (or decreases, respectively) with time as shown in Figure 7(d). From an epidemiological perspective, human leptospirosis infection can be minimized by reducing the number of infected individuals significantly using treatment control effort on infected individuals.

### 5.3. Effect of the Mortality Rate of Rodents (*μ*_*v*_)

From Figures 5(b), 6(c), and 7(d), increasing the number of susceptible rodents depends on the reduction of the parameters *β*_1_, *β*_3_, and *δ* on susceptible humans, susceptible rodents, and infected individuals, respectively. However, reducing these parameters may cause an increase in the total number of rodent population slowly (as can be seen in the figures). Thus, the control mechanism for growth of the rodent population (for instance, rodenticide) should be implemented to reduce the total number of rodent population. The effect of mortality rate of rodents *μ*_*v*_ in human, rodent, and bacterial population is illustrated in this section by using the different values of *μ*_*v*_ as *μ*_*v*_ = 0.001, *μ*_*v*_ = 0.0029, *μ*_*v*_ = 0.0059, *μ*_*v*_ = 0.009, and *μ*_*v*_ = 0.014. It can be observed, from Figures 8(b)–8(f), that the number of infected individuals, the total number of rodents (*S*_*V*_ + *I*_*v*_ + *R*_*V*_), and the size of bacterial population decrease as *μ*_*v*_ increases. Conversely, decreasing the mortality rate of rodents decreases the number of susceptible humans as shown in Figure 8(a).

The article "A Mathematical Model Analysis for the Transmission Dynamics of Leptospirosis Disease in Human and Rodent Populations" was published in 2022. Journal: Comput Math Methods Med.

Therefore, controlling the major direct zoonotic infections in a human population depends on the reduction of animal reservoirs, as in the case of leptospirosis infection. Reduction of the rodent population may also reduce the number of human infections as well as the concentration of *Leptospira interrogans* in the environment. Thus, the rodent born leptospirosis infections of humans can be controlled by implementing rodents' reduction mechanism. Further, since *R*_0_ ≈ 2.8552 > 1, all trajectories of the model solutions eventually move towards the unique positive *E*_*l*_^∗^. Thus, it should be intensified to use optimal efforts on interventions to eliminate the disease in the infected population as much as possible.

## 6. Conclusion

In this work, we presented and analyzed a deterministic mathematical model for the transmission process of leptospirosis disease, which includes human, vector (rodent), and bacterial populations. Firstly, the qualitative properties of the model are studied. Based on the next-generation matrix approach, the basic reproduction number (*R*_0_) of the formulated model is computed to perform sensitivity analysis of the model parameters. From the stability analysis of the model, we found that the disease-free equilibrium (DFE) is globally asymptotically stable if *R*_0_ < 1 and unstable otherwise. The local stability of an endemic equilibrium is performed based on the general center manifold theory, and EE is locally asymptotically stable when *R*_0_ < 1. The model exhibits forward bifurcation. This shows that the leptospirosis disease can be eradicated in infected population as long as when *R*_0_ < 1. The most sensitive parameters for *R*_0_ are *Λ*, *Π*, *μ*, *β*_1_, *β*_3_, *μ*_*v*_, and *δ*, among other parameters. This illustrates that minimizing the number of infected individuals depends on the reduction of *β*_1_ on susceptible individuals and the increase of recovery rate *δ*. This shows that minimizing the human infection depends on the reduction of *β*_3_ on susceptible vectors and the increase of mortality rate of rodents *μ*_*v*_. Epidemiological implications of this illustrate that preventive and control efforts should be targeted on the parameters *β*_1_, *β*_3_, and *μ*_*v*_ to reduce the burden of the disease in human populations since it is not reasonable ethically or biologically to use the death rate of humans as a control measure. Finally, the model is simulated to show the changing effects of the most influencing parameters on the disease expansion as well as the stability behaviors of the steady states. From graphical stability behavior of EE, all trajectories of the model solutions eventually move to the unique EE for *R*_0_ ≈ 2.8552 > 1. In this case, the disease persists in the population. On the other hand, all trajectories of the model solutions gradually move towards the DFE for *R*_0_ < 1. The biological implication of this shows that the disease will die from a community as long as when the basic reproduction number of the model is less than unity. Therefore, the value of *R*_0_ should be reduced as much as possible to eradicate the disease rapidly in an infected population. Moreover, our numerical results of the model demonstrate that reducing the transmission of human leptospirosis infection can be achieved by implementing the presentation and control interventions. Thus, our study recommends the following intervention efforts to minimize the risk factors and control the disease infection that should be implemented in human, rodent, and bacterial populations in an infected community:

- Reduce the rodent population using rodenticide or resource reduction. Implementation of this intervention also reduces the shedding rate of leptospire into the environment
- Prevention interventions on susceptible humans. Avoid contact with infected rodents and rodents urine-contaminated environment (floodwater, lakes, rivers, or soil) using an appropriate personal protective equipment (PPE) such as wearing rubber boots, waterproof dressings to cover wounds or skin, goggles, and rubber gloves as well as maintaining good personal hygiene. These practices will minimize the acquisition of the infection in the community
- Use the treatment control on infected individuals. Although the leptospirosis infection shows nonfixed symptoms and signs initially, its clinical manifestation can be detected by microbiological laboratory tests. This control mechanism can minimize the expansion of the disease by treating infected individuals through antibiotics that are recommended for treatment of the disease in the infected population following clinical rules
- Increase mortality rate of *Leptospira interrogans* in environment (especially, urban slum environment) using appropriate environmental modifications

These clinical interpretations (interventions) can be implemented by heightening the awareness of public health-care sectors on the spread and impacts of the disease on human health and by providing information for infected populations to use an effort to minimize the risk factors of the disease through intensifying successive education (or training) on the disease. However, to illustrate the effectiveness and cost-effectiveness of these intervention efforts an optimal control intervention should be studied.

The article "A Mathematical Model Analysis for the Transmission Dynamics of Leptospirosis Disease in Human and Rodent Populations" was published in 2022. Journal: Comput Math Methods Med.

## Figures and Tables

**Figure 1:** Compartmental flow diagram of leptospirosis disease transmission.

**Figure 2:** Forward bifurcation.

**Figure 3:** Plots showing the stability behavior of EE, *E*_1_^∗^ = (47.668,6.5229,5.3154,4.2571,628.6425,34.9632,26.0494,146.2314) of the model (3) as *t* varies.

**Figure 4:** Plots showing the stability behavior of DFE, *ε*_0*l*_^∗^ = (300,0, 0, 0, 571.4,0, 0, 0) of the model (3) as time changes.

**Figure 5:** Plots showing the sensitivity of model (3) using different values of *β*_1_.

**Figure 6:** Plots showing the sensitivity of model (3) using different values of *β*_3_.

**Figure 7:** Plots showing the sensitivity of model (3) using different values of *δ*.

**Figure 8:** Plots showing the sensitivity of model (3) using different values of *μ*_*v*_.

**Table 1:** Description of variables of the leptospirosis disease model.

Variable	Description
*S*_*h*_(*t*)	The susceptible individuals; individuals who are healthy but can be infected
*E*_*h*_(*t*)	Latently infected individuals; individuals having the disease but not showing the symptoms
*I*_*h*_(*t*)	The infectious individuals that are showing symptoms of the disease and can transmit disease to others
*R*_*h*_(*t*)	Those that have recovered from the disease and have got temporary immunity
*S*_*v*_(*t*)	Susceptible rodents
*I*_*v*_(*t*)	Infected rodents
*R*_*v*_(*t*)	Rodents that are recovered from the disease
*B*_*l*_	Leptospirosis causing bacterial population

**Table 2:** Description of parameters of the leptospirosis disease model.

Parameter	Description
*Λ*	The recruitment rate of susceptible humans
*Π*	The recruitment rate of susceptible rodents
*β*_1_	The transmission coefficient of the disease from infected rodents to susceptible humans
*β*_2_	The transmission rate of infection from environment to human
*β*_3_	The transmission rate of infection from infectious individuals to susceptible rodents
*γ*	The disease waning immunity for humans
*μ*	The natural death rate of the human population
*μ*_*v*_	The natural death rate of rodent population
*μ*_*b*_	The natural death rate of leptospirosis causing bacteria population
*θ*	The rate of the exposed human move to infected class
*α*	The death rate due to the disease infection
*δ*	The recovery rate from symptomatic infectious
*ρ*	The disease waning immunity for rodents
*σ*	Rate of recovery from leptospirosis rodent infection
*κ*	The concentration of pathogenic population in environment
*τ*_1_	The rate of increase of bacteria by *I*_*h*_
*τ*_2_	The rate of increase of bacteria by *I*_*v*_

The article "A Mathematical Model Analysis for the Transmission Dynamics of Leptospirosis Disease in Human and Rodent Populations" was published in 2022. Journal: Comput Math Methods Med.

**Table 3:** Sensitivity indices of *R*_0_ to each of the parameter values.

Parameter	Value	Sensitivity index
*Λ*	0.27	0.5421
*μ*_*v*_	0.0029	−0.0306
*μ*	0.0009	−0.0058
*Π*	2	0.4579
*β*_3_	0.0007	0.4579
*σ*	0.064	−0.438
*β*_1_	0.00033	0.4167
*δ*	0.072	−0.3457
*α*	0.04	−0.1921
*β*_2_	0.0815	0.5
*κ*	10000	−0.1254
*τ*_1_	0.06	0.0842
*τ*_2_	0.2	0.0412
*μ*_*b*_	0.05	−0.1254
*θ*	0.092	0.0004879

**Table 4:** Description of parameter values used in the simulations.

Parameter	Description	Value	Unit	Source
*Λ*	The recruitment rate of susceptible humans	*μ* × *N*0	Humans day^−1^	Assumed
*Π*	The recruitment rate of susceptible rodents	2	Rodents day^−1^	[5]
*β*_1_	The transmission coefficient between *S*_*h*_ and *I*_*v*_	0.00033	(Rodents day)^−1^	Assumed
*β*_2_	The transmission coefficient between *S*_*h*_ and *B*_*b*_	0.0815	Day^−1^	Assumed
*β*_3_	The transmission coefficient between *S*_*v*_ and *I*_*h*_	0.0007	(Humans day)^−1^	Assumed
*μ*	The natural death rate of susceptible humans	0.0009	Day^−1^	[29]; [5]
*α*	The disease-related death rate of humans	0.04	Day^−1^	Assumed
*θ*	The rate at which latently infected individual transfer to infectious	0.092	Day^−1^	[30]
*γ*	Leptospirosis disease waning immunity from *R*_*h*_	0.089	Day^−1^	[31]
*δ*	The rate at which infectious individual transfer to human recovery class	0.072	Day^−1^	Assumed
*σ*	The rate of recovery from infectious rodent	0.064	Day^−1^	Assumed
*ρ*	Leptospirosis disease waning immunity from *R*_*v*_	0.083	Day^−1^	Assumed
*μ*_*v*_	The natural death rate of the rodents	0.0029	Day^−1^	[29]
*μ*_*b*_	The natural death rate of the bacteria	0.05	Day^−1^	[6]
*τ*_1_	The rate of increase of bacterial population due to *I*_*h*_	0.06	$\frac{\text{No}.\text{of pathogen}}{\text{humans day}}$	Assumed
*τ*_2_	The rate of increase of bacterial population due to *I*_*v*_	0.2	$\frac{\text{No}.\text{of pathogen}}{\text{rodents day}}$	Assumed
*κ*	The concentration of pathogenic population	10000	No.of pathogen	Assumed

## Data Availability

The numerical data used to support the findings of this study have been taken from previously published articles and cited in the Table 4 of this paper. These published articles are also cited at relevant places within the text as references.

## Abbreviations

WHO: World Health Organization
CDC: Centers for Disease Control and Prevention
DFE: Disease-free equilibrium
EE: Endemic equilibrium
ODE: Ordinary differential equation
SIR: Susceptible-infected-removed
SEIR: Susceptible-exposed-infected-removed.
